The article "Decision algorithm for educational institute selection with spherical fuzzy heronian mean operators and Aczel-Alsina triangular norm" was retracted in 2025. Reason: concerns about the citations.

# Decision algorithm for educational institute selection with spherical fuzzy heronian mean operators and Aczel-Alsina triangular norm

**DOI:** 10.1016/j.heliyon.2024.e28383

**Published:** 2024-03-26

**Authors:** Abrar Hussain, Kifayat Ullah, Sajid Latif, Tapan Senapati, Sarbast Moslem, Domokos Esztergar-Kiss

**Affiliations:** a Department of Mathematics, Riphah International University Lahore Campus, 54000, Lahore, Pakistan; b School of Mathematics and Statistics, Southwest University, Chongqing, People's Republic of China; c School of Architecture Planning and Envirinmental Policy, University College of Dublin, D04 V1W8, Belfield, Dublin, Ireland; d Department of Transport Technology and Economics, Faculty of Transportation Engineering and Vehicle Engineering, Budapest University of Technology and Economics, Műegyetem Rkp. 3, Budapest, Hungary

**Keywords:** Spherical fuzzy set values, Aczel Alsina aggregation operations, Heronian mean models, And decision support system

## Abstract

This article presents a novel study of spherical fuzzy sets (SFSs), a more comprehensive framework of intuitionistic fuzzy sets and picture fuzzy sets. The SFS allows the decision-makers (DMs) to cope with complicated and insufficient information during the aggregation process. The Heronian mean (HrM) model theory is also utilized to express correlation among different input arguments or characteristics. Recently, the theory of Aczel Alsina triangular norms gained a lot of attention from various research scholars and has many capabilities to provide smooth approximations during decision analysis. In this article, we developed some appropriate operations of Aczel Alsina t-norms and t-conorms in light of spherical fuzzy (SF) information. We develop new mathematical ways to look at SF data to keep clarity and sufficient information. These are the SF Aczel Alsina Heronian mean (SFAAHrM) and SF Aczel Alsina weighted Heronian mean (SFAAWHrM) operators. Furthermore, we also present a list of new strategies based on Aczel Alsina operations, such as SF Aczel Alsina geometric Heronian mean (SFAAGHrM) and SF Aczel Alsina weighted geometric Heronian mean (SFAAWGHrM) operators. Some notable properties are also characterized to show the validity and effectiveness of our derived mathematical approaches. Considering our derived strategies, an algorithm for the multiple attribute decision-making (MADM) problem is established to resolve complicated real-life applications. A numerical example presents the compatibility of derived approaches and provides a solid mechanism to improve the performance of educational institutes. A comparison technique is also demonstrated to show the applicability and consistency of diagnosed approaches by contrasting the findings of pioneered approaches with existing methodologies.

## 1 Introduction

The MADM technique evaluates a reliable, optimal option based on particular criteria or attributes. This advanced strategy of the decision-making process allows the decision-maker to identify an appropriate individual based on specific preferences. The decision-maker faces a lot of complexities and challenges due to incomplete or redundant information about human opinion. To address such situations, Zadeh [1] proposed the fuzzy set (FS) to tackle ambiguous and uncertain information about human opinion. An FS defines the truth membership value (TMV) of every element of the universal set within the condition [0,1] to characterize the unpredictability of the information. An element may belong to the universal set or not in a crisp set. So, it was not a very valuable tool to describe human views broadly. FS is a more expandable system rather than the crisp set because it contains all the values in [0,1]. Moreover, Atanassov [2] invented the idea of the intuitionistic fuzzy set (IFS), which enlarged the study of FS by including the falsity membership value (FMV) along with the TMV within the condition [0,1] which is the best way to express the human point of view positively and negatively. According to the IFS model, only some specific information in the form of duplets is permitted such that 0≤₥≤1 and 0≤n≤1. IFS fulfills the condition that 0≤₥+n≤1 provides flexibility in selecting the TMV and FMV. The sum of TMV and FMV occasionally exceeds the limit of [0,1]. Due to these restrictions, the IFS cannot be employed in many decision-making (DM) situations when 0≤₥+n≤1 exceeds the limit [0,1]. To deal with such circumstances, Yager [3,4] developed the ideology of the Pythagorean fuzzy set (PyFS), which allows $0\leq {₥}^{2}+n^{2}\leq 1$ and explains its applications. However, in some cases, when the sum of the square of TMV and FMV surpasses [0,1], PyFS is unable to explain such situations. To contend with such situations, Yager [5] put forward the concept of q-rung orthopair fuzzy set (q-ROFS) with the restriction $0\leq {₥}^{q}+n^{q}\leq 1$ providing extensive information in dealing with inconsistencies. The IFS and PyFS are the particular cases of q-ROFS. The boundary of assessment information described by the TMV and FMV also becomes larger when the parameter q value increases in q-ROFS. In q-ROFS, the TMV and FMV represent the parts that belong to and do not belong to a given set, respectively, while the remaining portion is referred to as uncertainty or hesitation value. It occurs in some circumstances involving choices (such as casting votes), and people find new ways to express their opinions. Coung [6] suggested the notion of a picture fuzzy set (PFS) in the form (₥,ѯ,n) where the elements in the triplet represent TMV, abstinence membership value (AMV), and FMV with the restriction 0≤₥+ѯ+n≤1, and the refusal degree is defined as Ŗ=1−(₥+ѯ+n). The PFS hypothesis is ineffective in many experimental circumstances. It is noticed that the condition 0≤₥+ѯ+n≤1 in PFS makes us incapable to allocate each value ₥,ѯ, and n on their own. To overcome this concern, Mahmood et al. [7] introduced the ideology of a spherical fuzzy set (SFS) with the restriction $0\leq {₥}^{2}+{ѯ}^{2}+n^{2}\leq 1$ such that TMV, AMV, and FMV lie [0,1] significantly broadens the PFS range. However, using SFS theory, there may be some problems. Mahmood et al. [8] further used the idea of SFS and gave its approach to DM and medical diagnosis problems. But it is not still more useful for a few triplets. This assisted in the concept of a T-spherical fuzzy set (T-SFS). Ullah et al. [9] utilized the term T-SFS, which is a generalization of SFS and provides a wide range of solutions to real-world issues.

The theory of the decision-making process is utilized to evaluate an appropriate optimal option under consideration of different criteria. Several research scholars classified different algorithms and evaluated multiple applications of real-life challenges. The AOs are several efficient aggregation tools that investigate uncertainty in human opinions. First, Xu et al. [[10], [11], [12]] expanded the idea of basic arithmetic and geometric aggregation tools by using the product t-norm (T-NM) and probabilistic t-conorms (TC-NM). Several mathematicians used different aggregation techniques to illustrate inadequate and dubious information during decision-making procedures. There are many types of T-NM and TC-NM, which are the modifications of triangular norms such as Lukasiewicz [13] T-NM and TC-NM, Drastic [14] T-NM and TC-NM, Archimedean [15] and Frank [16] T-NM and TC-NM. Riaz and Farid [17] illustrated advanced decision-making approaches and established new strategies using the basic operations of relatively aggregation tools. Seikh and Mandal [18] anticipated new mathematical methods for q-rung orthopair fuzzy theory by utilizing the properties of Archimedean t-norms. Wang [19] put forward the theory of 2-tuple fuzzy linguistic sets for the evaluation of real-life situations under the system of the MAGDM problem. Assessing social trust propagation is another strategy for solving the decision-making problem that Liu et al. [20] demonstrated. Hussain et al. [21] grouped different tourist spots and devised an excellent structure for boosting the economy of any area. Biswas and Deb [22] applied the basic ideas of PyF information to show how reliable Schweizer Sklar aggregation operators are. Senapati et al. [23], who investigated a suitable source of transport under the system of decision-making problems, developed the idea of sustainable transportation-sharing practices. Akram et al. [24] built on Muirhead's idea of mean aggregation tools, using the theory of 2-tuple linguistic sets to show how different things are related. Ali and Naeem [25] established an advanced decision-making approach with the help of unknown weight information. Akram and Bibi [26] found a novel approach for decision analysis under the 2-tuple linguistic Fermatean fuzzy theory system. Kakati et al. [71] anticipated an unknown Fermatean fuzzy Archimedean Heronian mean-based model for evaluating urban transport sustainability.

Ullah [27] studied specific applications of the decision-making problems in light of Maclurin symmetric mean aggregation tools. Dhumras and Bajaj [28] established some dominant approaches to picture fuzzy theory with the characteristics of hypersoft sets. Bansal et al. [29] anticipated new mathematical approaches by utilizing some particular features of the hypersoft set by incorporating the system of T-spherical fuzzy situations. An innovative approach for decision analysis, like the WASPAS and AHP methods based on the q-rung orthopair picture fuzzy theory, was presented by Dhumras and Bajaj [30]. A novel approach to picture fuzzy information and new mathematical approaches based on Frank t-norms established by Seikh and Mandal [31]. Mandal and Seikh [32] also resolved an application of waste management under the system of interval-valued SF theory with advanced decision-making problems. Moslem [72] proposed a novel model based on an analytic hierarchy process with fuzzy sets and parsimonious information preferences to facilitate the urban transport system. However, Moslem et al. [73] presented the spherical fuzzy analytical hierarchy process with Kendall's agreement to estimate the riskiest driver behaviour factors related to road safety.

Firstly, Beliakov et al. [33] introduced a robust concept of HrM operators to express relationships among different input arguments. With time, several mathematicians explored the theory of HrM operators under other fuzzy circumstances. Sỳkora [31] also developed specific approaches by generalizing the theory of HrM operators. Yu [34] proposed some particular methodologies of the HrM operators based on intuitionistic fuzzy information. Khan et al. [35] demonstrated the theory of cubic Schweizer Sklar aggregation tools using unknown weight vectors. Some reliable operations of interactional aggregation tools developed by Wang and Zhang [36] are the modified version of basic operations. Hussain et al. [37] evaluated a particular solar panel using the theory of HrM operators under an IF information system. Some specific approaches of the HrM operators based on hesitant q-ROF circumstances were also developed by Sarkar et al. [38]. Li and Wei [39] combined a mixture of two different notions, such as HrM and PyF information, to illustrate sustainable supplier enterprises. Wei et al. [40] modified two other concepts of the HrM and GHrM operators under the system of q-ROF information to solve real-life issues. Hussain et al. [41] presented new approaches to Hamy mean operators by exploring the characteristics of Dombi t-norms under the system of SF environment. Wei et al. [42] defined interrelationships among different objects using the theory of HrM operators and established decision-making approaches. Several mathematicians utilized the concepts of HrM aggregation tools to express correlations among other arguments [[43], [44], [45]].

Aczel and Alsina [46] introduced a family of robust aggregation tools by generalizing the theoretical concepts of triangular norms. The basic operations of Aczel Alsina T-NM and TC-NM are well-known aggregations that provide a smooth approximation during the aggregation process. Aczel Alsina T-NM and TC-NM operations are attractive due to their flexibility, and several mathematicians have utilized the theory of Aczel Alsina aggregation tools in different fuzzy circumstances. Senapati et al. [47] resolved an application of real-life situations under the system of intuitionistic fuzzy information. Sarfraz et al. [48] employed the notion of prioritized AOs by using basic operations of Aczel Alsina aggregation tools. Hussain et al. [49] anticipated new approaches of PyFSs to evaluate a notable candidate for a multinational company. Naeem et al. [50] developed new techniques based on Aczel Alsina aggregation tools under the PFS system. Hussain et al. [[51], [52], [53]] also explored the theory of Aczel Alsina expressions and derived new mathematical strategies for solving real-life applications. Riaz et al. [54] discussed the theory of Aczel Alsina aggregation tools, considering the spherical fuzzy information.

Although we studied a lot of benefits of the above-discussed research works, some weaknesses and limitations were also found by the decision-maker during the decision analysis. Sometimes, the aforementioned mathematical approaches can only be insufficient because the theory of FSs, IFSs, and PFSs are limited and narrow in their structural behaviour. To serve this situation, the theory of SFSs is the extended version of IFSs and PFSs, which capture three different components of human opinions with the sum of the square of TMV, AMV, and FMV limited on the interval [0, 1]. Many computational mathematical models like Hamy mean, Symmetric mean, Bneferroni mean, and many other strategies are used to aggregate vague type information. All discussed strategies and models have some drawbacks due to the restricted and limited approach of the parameters. On the other hand, the concepts of the HrM operators are utilized to express the interrelationship among different arguments through the various parameters and variables. Experts may achieve realistic and authentic results during decision-making by varying these parameters and variables. We also studied the nature of different T-NM and TC-NM, such as Frank T-NM and TC-NM, Dombi T-NM and TC-NM, and Einstein T-NM and TC-NM. Finally, we concluded that Aczel Alsina aggregation tools are more efficient and provide a smooth approximation during the decision-making process. These days, Aczel Alsina aggregation tools are an attractive research topic, and numerous mathematicians explore the theoretical concepts of Aczel Alsina aggregation tools in different fuzzy circumstances. We see no one working on SFSs under the system of HrM models to tackle redundant information of human opinion. Considering the significance of HrM models and Aczel Alsina aggregation operations, we explore new approaches to investigate inherent inadequate and uncertain information. The critical components of this research work are characterized as follows.

i. To handle uncertain and ambiguous information about human opinion, we expose the theory of SFS with some reliable features and characteristics.
ii. Motivated by the significance of the SF environment, some realistic operational laws are also present in the light of SF information.
iii. To develop a list of new approaches based on Aczel Alsina aggregation tools, including SFAAHrM, SFAAWHrM, SFAAGHrM, and SFAAWGHrM operators. Some special cases and reliable properties of our invented approaches are also discussed.
iv. The MADM technique is also employed to resolve real-life situations under the system of SF information. To find the applicability and effectiveness of derived mathematical approaches, we gave an appropriate numerical example to enhance the performance of the educational institutes under some particular characteristics.
v. Through the comparison method, we measured the efficacy of our developed operators by contrasting the findings of pioneered approaches with existing mathematical approaches that exist in the literature.

This article is divided into the following parts: Section 2 covers basic notions of SFSs and their related basic operations necessary to improve current research work. Demonstrates some appropriate operations of Aczel Alsina aggregation tools under the system of SF information in Section 3. In section 4, we developed a list of new approaches by exploring the theoretical concepts of HrM operators, such as SFAAHrM and SFAAWHrM operators. Furthermore, another list of new methods is based on GHrM operators using Aczel Alsina aggregation tools such as SFAAGHrM and SFAAWGHrM operators. To demonstrate the viability of our derived techniques, we constructed an algorithm for an efficient decision-making problem in section 6. To see the advantages and consistency, we gave a comparison model to contrast the findings of our derived strategies with existing techniques in section 7. Some specific remarks on the conclusion are presented in Section 8.

## 2 Preliminaries

Now, we will express some basic notions of the Triangular norms, SFSs, and their related fundamental rules, which are essential for improving this article. All symbols with their meanings are shown in Table 1.

Definition 1 [55] A mapping T:[0,1]×[0,1]⟶[0,1] is referred to as T-NM ∀ε,υ,r∈[0,1] if it meets the listed properties such as symmetry, monotonicity, associativity, and one identity element.

i.T(ε,υ)=T(υ,ε).
ii.T(ε,υ)≤T(ε,r) if υ≤r.
iii.T(ε,T(υ,r))=T(T(ε,υ),r).
iv.T(ε,1)=ε.

Definition 2 [55] A mapping S∶[0,1]×[0,1]⟶[0,1] is referred to as TC-NM if it meets the listed properties such as symmetry, monotonicity, associativity, and zero identity element.

i.S(ε,υ)=S(υ,ε).
ii.S(ε,υ)≤S(ε,r) if υ≤r.
iii.S(ε,S(υ,r))=S(S(ε,υ),r).
iv.S(ε,0)=ε.

**Table 1:** Symbols and their meanings.

Symbols	Meanings	Symbols	Meanings
₡	Parametric value of Aczel Alsina	k	Score function
R	Universal set	T	Accuracy function
ӽ	Element of Universal set	⍹	Weight vector
₥	truth membership value	Ⱥ	Alternative
ѯ	abstinence membership values	ŧ	Attribute
n	falsity membership value	℟	Decision matrix
$T_{A}^{₡}$	Aczel Alsina t-norm	$S_{A}^{₡}$	Aczel Alsina t-conorm
Ῠ	Spherical fuzzy value	Ŗ	refusal degree
T	t-norm	S	t-conorm

For all ε,υ,r∈[0,1].

Definition 3 [46] The term ${T_{A}^{₡}}_{₡\in \left[0,1\right]}$ of Aczel Alsina T-NM is defined as:

$$T_{A}^{₡}\left(\varepsilon ,\upsilon \right)=\left\{ \begin{array}{cc} \begin{array}{c} T_{D}\left(\varepsilon ,\upsilon \right)\\ min\left(\varepsilon ,\upsilon \right)\\ e^{-{\left({\left(-\log\;\varepsilon \right)}^{₡}+{\left(-\log\;\upsilon \right)}^{₡}\right)}^{\frac{1}{₡}}} \end{array} & \begin{array}{c} if\;₡=0\\ if\;₡=\infty \\ \text{otherwise} \end{array} \end{array}\right.$$

The term ${S_{A}^{₡}}_{₡\in \left[0,1\right]}$ of Aczel Alsina TC-NM is defined as:

$$S_{A}^{₡}\left(\varepsilon ,\upsilon \right)=\left\{ \begin{array}{cc} \begin{array}{c} S_{D}\left(\varepsilon ,\upsilon \right)\\ \max\left(\varepsilon ,\upsilon \right)\\ 1-e^{-{\left({1-\left(-\log\left(1-\varepsilon \right)\right)}^{₡}+{\left(-\log\left(1-\upsilon \right)\right)}^{₡}\right)}^{\frac{1}{₡}}} \end{array} & \begin{array}{c} \text{if}\;₡=0\\ \;\text{if}\;₡=\infty \\ \;\text{otherwise} \end{array} \end{array}\right.$$

Definition 4 [56] For any universal set R and A be a PFS on the universal set. Then, it is defined as:

$$A=\left\{\left(ӽ,{₥}_{A}\left(ӽ\right),{ѯ}_{A}\left(ӽ\right),n_{A}\left(ӽ\right)\right)|ӽ\in R\right\}$$

Where the mappings are ${₥}_{A}\left(ӽ\right):R\to \left[0,1\right]\text{,}$ ${ѯ}_{A}\left(ӽ\right):R\to \left[0,1\right]$ and $n_{A}\left(ӽ\right):R\to \left[0,1\right]$ indicate the truth membership value (TMV), abstinence membership values (AMV), and falsity membership value (FMV) of ӽ in R, respectively. A PFS must fulfill the following conditions:

$$0\leq {₥}_{A}\left(ӽ\right)+{ѯ}_{A}\left(ӽ\right)+n_{A}\left(ӽ\right)\leq 1$$

Definition 5 [8] Let R be a universal set and A be an SFS on a universal set. Then, an SFS is defined as:

$$A=\left\{\left(ӽ,{₥}_{A}\left(ӽ\right),{ѯ}_{A}\left(ӽ\right),n_{A}\left(ӽ\right)\right)|ӽ\in R\right\}$$

Where are the mappings ${₥}_{A}\left(ӽ\right):R\to \left[0,1\right]\text{,}$ ${ѯ}_{A}\left(ӽ\right):R\to \left[0,1\right]$ and $n_{A}\left(ӽ\right):R\to \left[0,1\right]$ with TMV, AMV, and FMV signifying their membership value of ӽ in R, respectively. A SFS must fulfill the following conditions:

$$0\leq {{₥}_{A}}^{2}\left(ӽ\right)+{{ѯ}_{A}}^{2}\left(ӽ\right)+{n_{A}}^{2}\left(ӽ\right)\leq 1$$

The refusal degree is given as ${Ŗ}_{A}\left(Ῠ\right)=1-\left(\sqrt{{{₥}_{A}}^{2}\left(ӽ\right)+{{ѯ}_{A}}^{2}\left(ӽ\right)+{n_{A}}^{2}\left(ӽ\right)}\right)$. For convention, we say that Ῠ=(₥(ӽ),ѯ(ӽ),n(ӽ)) is known as spherical fuzzy value (SFV).

Definition 6 [54] Let ${Ῠ}_{1}=\left\{\left(ӽ,{₥}_{1}\left(ӽ\right),{ѯ}_{1}\left(ӽ\right),n_{1}\left(ӽ\right)\right)|ӽ\in R\right\}$ and ${Ῠ}_{2}=\left\{\left(ӽ,{₥}_{2}\left(ӽ\right),{ѯ}_{2}\left(ӽ\right),n_{2}\left(ӽ\right)\right)|ӽ\in R\right\}$ be the two SFVs. Then, the basic operations of union, intersection and compliment are termed as:

i.${Ῠ}_{1}\cup {Ῠ}_{2}=\left\{\max\left({₥}_{1}\left(ӽ\right),{₥}_{2}\left(ӽ\right)\right),min\left({ѯ}_{1}\left(ӽ\right),{ѯ}_{2}\left(ӽ\right)\right),min\left(n_{1}\left(ӽ\right),n_{2}\left(ӽ\right)\right)\right\}$.
ii.${Ῠ}_{1}\cap {Ῠ}_{2}=\left\{min\left({₥}_{1}\left(ӽ\right),{₥}_{2}\left(ӽ\right)\right),\max\left({ѯ}_{1}\left(ӽ\right),{ѯ}_{2}\left(ӽ\right)\right),\max\left(n_{1}\left(ӽ\right),n_{2}\left(ӽ\right)\right)\right\}$.
iii.${{Ῠ}_{1}}^{c}=\left(n_{1}\left(ӽ\right),{ѯ}_{1}\left(ӽ\right),{₥}_{1}\left(ӽ\right)\right)$.
iv.${Ῠ}_{1}={Ῠ}_{2}$ if and only if ${Ῠ}_{1}\subseteq {Ῠ}_{2}$ and ${Ῠ}_{2}\subseteq {Ῠ}_{1}$.

Definition 7 [54] Let ${Ῠ}_{1}=\left\{\left(ӽ,{₥}_{1}\left(ӽ\right),{ѯ}_{1}\left(ӽ\right),n_{1}\left(ӽ\right)\right)|ӽ\in R\right\}$ and ${Ῠ}_{2}=\left\{\left(ӽ,{₥}_{2}\left(ӽ\right),{ѯ}_{2}\left(ӽ\right),n_{2}\left(ӽ\right)\right)|ӽ\in R\right\}$ be the two SFVs in R and ѯ>0. Then, some appropriate operations of SFVs are expressed as follows:

i.${Ῠ}_{1}⊕{Ῠ}_{2}=\left(\sqrt{{{₥}_{1}}^{2}+{{₥}_{2}}^{2}-{{₥}_{1}}^{2}{{₥}_{2}}^{2}},{ѯ}_{1}{ѯ}_{2},n_{1}n_{2}\right)$.
ii.${Ῠ}_{1}⊗{Ῠ}_{2}=\left({₥}_{1}{₥}_{2},\sqrt{{{ѯ}_{1}}^{2}+{{ѯ}_{2}}^{2}-{{ѯ}_{1}}^{2}{{ѯ}_{2}}^{2}},\sqrt{{n_{1}}^{2}+{n_{2}}^{2}-{n_{1}}^{2}{n_{2}}^{2}}\right)$.
iii.$ѯῨ=\left(\sqrt{1-{\left(1-{\left(₥\right)}^{2}\right)}^{ѯ}},{\left(ѯ\right)}^{ѯ},{\left(n\right)}^{ѯ}\right)$.
iv.${Ῠ}^{ѯ}=\left({\left(₥\right)}^{ѯ},\sqrt{1-{\left(1-{\left(ѯ\right)}^{2}\right)}^{ѯ}},\sqrt{1-{\left(1-{\left(n\right)}^{2}\right)}^{ѯ}}\right)$.

Definition 8 [54] Let ${Ῠ}_{1}=\left\{\left(ӽ,₥\left(ӽ\right),ѯ\left(ӽ\right),n\left(ӽ\right)\right)|ӽ\in R\right\}$, ${Ῠ}_{2}=\left\{\left(ӽ,{₥}_{1}\left(ӽ\right),{ѯ}_{1}\left(ӽ\right),n_{1}\left(ӽ\right)\right)|ӽ\in R\right\}$ and ${Ῠ}_{2}=\left\{\left(ӽ,{₥}_{2}\left(ӽ\right),{ѯ}_{2}\left(ӽ\right),n_{2}\left(ӽ\right)\right)|ӽ\in R\right\}$ are three SFVs in R and ѯ>0, so we have:

i.${Ῠ}_{1}⊕{Ῠ}_{2}={Ῠ}_{2}⊕{Ῠ}_{1}$.
ii.${Ῠ}_{1}⊗{Ῠ}_{2}={Ῠ}_{2}⊗{Ῠ}_{1}$.
iii.$ѯ\left({Ῠ}_{1}⊕{Ῠ}_{2}\right)=ѯ{Ῠ}_{1}⊕ѯ{Ῠ}_{2}$.
iv.${\left({Ῠ}_{1}⊗{Ῠ}_{2}\right)}^{ѯ}={{Ῠ}_{1}}^{ѯ}⊗{{Ῠ}_{2}}^{ѯ}\text{,}$ ѯ≥0.
v. ${ѯ}_{1}Ῠ⊕{ѯ}_{2}Ῠ=\left({ѯ}_{1}+{ѯ}_{2}\right)Ῠ$, ${ѯ}_{1},{ѯ}_{2}\geq 0$.
vi. ${Ῠ}^{{ѯ}_{1}}⊗{Ῠ}^{{ѯ}_{2}}={Ῠ}^{{ѯ}_{1}+{ѯ}_{2}}$, ${ѯ}_{1},{ѯ}_{2}\geq 0$.

Definition 9 [57] For any Ῠ=(₥(ӽ),ѯ(ӽ),n(ӽ)) SFV in R. Then, score function k(Ῠ) and accuracy function T(Ῠ) are termed as follows:

$$k\left(Ῠ\right)=\frac{1}{3}\left(2+₥\left(ӽ\right)-ѯ\left(ӽ\right)-n\left(ӽ\right)\right),k\left(Ῠ\right)\in \left[0,1\right]$$

T(Ῠ)=₥(ӽ)−n(ӽ),T(Ῠ)∈[0,1]

Definition 10 Let ${Ῠ}_{ҏ}=\left({₥}_{ҏ}\left(ӽ\right),{ѯ}_{ҏ}\left(ӽ\right),n_{ҏ}\left(ӽ\right)\right),ҏ=1,2$ be the assemblage of SFVs in R. By using Definition 9 of the score function and accuracy function, we can compare SFVs.

i. If $k\left({Ῠ}_{1}\right)<k\left({Ῠ}_{2}\right)$ then, ${Ῠ}_{1}<{Ῠ}_{2}$.
ii. If $k\left({Ῠ}_{1}\right)>k\left({Ῠ}_{2}\right)$ then, ${\;Ῠ}_{1}>{Ῠ}_{2}$.
iii. If $k\left({Ῠ}_{1}\right)=k\left({Ῠ}_{2}\right)$ then:
  a. If $A\left({Ῠ}_{1}\right)<A\left({Ῠ}_{2}\right)$ then, ${Ῠ}_{1}<{Ῠ}_{2}$.
  b.If $A\left({Ῠ}_{1}\right)>A\left({Ῠ}_{2}\right)$ then, ${Ῠ}_{1}>{Ῠ}_{2}$.

Definition 11 [8] Let ${Ῠ}_{ҏ}=\left({₥}_{ҏ}\left(ӽ\right),{ѯ}_{ҏ}\left(ӽ\right),n_{ҏ}\left(ӽ\right)\right),ҏ=1,2,3,\ldots ,n$ be any assemblage of SFVs in R with corresponding weight vector ${⍹}_{ҏ}$ of ${Ῠ}_{ҏ}$ such that $\sum_{ҏ=1}^{n}{⍹}_{ҏ}=1$ and ${⍹}_{ҏ}>0$. Then, spherical fuzzy weighted averaging (SFWA) is defined as:

$$SFWA\left({Ῠ}_{1},{Ῠ}_{2},\ldots ,{Ῠ}_{n}\right)=\sum_{ҏ=1}^{n}{{⍹}_{ҏ}Ῠ}_{ҏ}$$

Definition 12 [8] Let ${Ῠ}_{ҏ}=\left({₥}_{ҏ}\left(ӽ\right),{ѯ}_{ҏ}\left(ӽ\right),n_{ҏ}\left(ӽ\right)\right),ҏ=1,2,3,\ldots ,n$ be any assemblage of SFVs in R with corresponding weight vector ${⍹}_{ҏ}$ of ${Ῠ}_{ҏ}$ such that $\sum_{ҏ=1}^{n}{⍹}_{ҏ}=1$ and ${⍹}_{ҏ}>0$. Then, spherical fuzzy weighted geometric (SFWG) is defined as:

$$SFWG\left({Ῠ}_{1},{Ῠ}_{2},\ldots ,{Ῠ}_{n}\right)=\prod_{ҏ=1}^{n}{\left({Ῠ}_{ҏ}\right)}^{{⍹}_{ҏ}}$$

Definition 13 [33,58] Let ${Ῠ}_{ҏ}=\left({₥}_{ҏ}\left(ӽ\right),{ѯ}_{ҏ}\left(ӽ\right),n_{ҏ}\left(ӽ\right)\right),ҏ=1,2,3,\ldots ,n$ be an assemblage of crisp numbers. Then, the Heronian mean (HrM) operator is defined as:

$${HrM}^{t,\varphi }\left({Ῠ}_{1},{Ῠ}_{2},\ldots ,{Ῠ}_{n}\right)={\left(\left(\frac{2}{n\left(n+1\right)}\right)\left(\sum_{i=1}^{n}\sum_{j=1}^{n}\left({Ῠ}_{i}^{t}⊗{Ῠ}_{j}^{\varphi }\right)\right)\right)}^{\frac{1}{t+\varphi }}$$

Where t,φ>0.

Definition 14 [34] Let ${Ῠ}_{ҏ}=\left({₥}_{ҏ}\left(ӽ\right),{ѯ}_{ҏ}\left(ӽ\right),n_{ҏ}\left(ӽ\right)\right),ҏ=1,2,3,\ldots ,n$ be any collection of crisp numbers. Then, the geometric Heronian mean (GHrM) operator is defined as:

$${GHrM}^{t,\varphi }\left({Ῠ}_{1},{Ῠ}_{2},\ldots ,{Ῠ}_{n}\right)=\frac{1}{t+\varphi }\prod_{i=1}^{n}\prod_{j=1}^{n}{\left({tῨ}_{i}⊕\varphi {Ῠ}_{j}\right)}^{\frac{2}{n\left(n+1\right)}}$$

Where t,φ>0.

## 3 Aczel Alsina aggregation operators based on spherical fuzzy values

In this section, some basic operations of the Aczel Alsina T-NM and TC-NM are characterized under the system of SF information.

Definition 15 Let ${Ῠ}_{ҏ}=\left({₥}_{ҏ}\left(ӽ\right),{ѯ}_{ҏ}\left(ӽ\right),n_{ҏ}\left(ӽ\right)\right),ҏ=1,2,3,\ldots ,n$ be any assemblage of SFVs in R. Then, some appropriate operational laws of Aczel Alsina aggregation tools based on SFVs are described as follows:

i.${Ῠ}_{1}⊕{Ῠ}_{2}=\left(\begin{array}{c} \sqrt{1-e^{-{\left({\left(-\log\left(1-{₥}_{1}^{2}\left(ӽ\right)\right)\right)}^{₡}+{\left(-\log\left(1-{₥}_{2}^{2}\left(ӽ\right)\right)\right)}^{₡}\right)}^{\frac{1}{₡}}}},\\ e^{-{\left({\left(-\log\left({ѯ}_{1}\left(ӽ\right)\right)\right)}^{₡}+{\left(-\log\left({ѯ}_{2}\left(ӽ\right)\right)\right)}^{₡}\right)}^{\frac{1}{₡}}},\\ e^{-{\left({\left(-\log\left(n_{1}\left(ӽ\right)\right)\right)}^{₡}+{\left(-\log\left(n_{2}\left(ӽ\right)\right)\right)}^{₡}\right)}^{\frac{1}{₡}}} \end{array}\right),₡\geq 1$.
ii.${Ῠ}_{1}⊗{Ῠ}_{2}=\left(\begin{array}{c} e^{-{\left({\left(-\log\left({₥}_{1}\left(ӽ\right)\right)\right)}^{₡}+{\left(-\log\left({₥}_{2}\left(ӽ\right)\right)\right)}^{₡}\right)}^{\frac{1}{₡}}},\\ \sqrt{1-e^{-{\left({\left(-\log\left(1-{ѯ}_{1}^{2}\left(ӽ\right)\right)\right)}^{₡}+{\left(-\log\left(1-{ѯ}_{2}^{2}\left(ӽ\right)\right)\right)}^{₡}\right)}^{\frac{1}{₡}}}},\\ \sqrt{1-e^{-{\left({\left(-\log\left(1-n_{1}^{2}\left(ӽ\right)\right)\right)}^{₡}+{\left(-\log\left(1-n_{2}^{2}\left(ӽ\right)\right)\right)}^{₡}\right)}^{\frac{1}{₡}}}} \end{array}\right),₡\geq 1$.
iii.$ѯῨ=\left(\begin{array}{c} \sqrt{1-e^{-{\left(ѯ{\left(-\log\left(1-{₥}^{2}\left(ӽ\right)\right)\right)}^{₡}\right)}^{\frac{1}{₡}}}},\\ e^{-{\left({ѯ\left(-\log\left(ѯ\left(ӽ\right)\right)\right)}^{₡}\right)}^{\frac{1}{₡}}},\\ e^{-{\left({ѯ\left(-\log\left(n\left(ӽ\right)\right)\right)}^{₡}\right)}^{\frac{1}{₡}}} \end{array}\right),₡\geq 1$.
iv.${Ῠ}^{ѯ}=\left(\begin{array}{c} e^{-{\left({ѯ\left(-\log\left(₥\left(ӽ\right)\right)\right)}^{₡}\right)}^{\frac{1}{₡}}},\\ \sqrt{1-e^{-{\left(ѯ{\left(-\log\left(1-{ѯ}^{2}\left(ӽ\right)\right)\right)}^{₡}\right)}^{\frac{1}{₡}}}},\\ \sqrt{1-e^{-{\left(ѯ{\left(-\log\left(1-n^{2}\left(ӽ\right)\right)\right)}^{₡}\right)}^{\frac{1}{₡}}}} \end{array}\right),₡\geq 1$.

Theorem 1 *For any three SFVs*${Ῠ}_{1}=\left\{\left(ӽ,₥\left(ӽ\right),ѯ\left(ӽ\right),n\left(ӽ\right)\right)|ӽ\in R\right\}$, ${Ῠ}_{2}=\left\{\left(ӽ,{₥}_{1}\left(ӽ\right),{ѯ}_{1}\left(ӽ\right),n_{1}\left(ӽ\right)\right)|ӽ\in R\right\}$*and*${Ῠ}_{2}=\left\{\left(ӽ,{₥}_{2}\left(ӽ\right),{ѯ}_{2}\left(ӽ\right),n_{2}\left(ӽ\right)\right)|ӽ\in R\right\}$*in*R*and*ѯ>0. *We have*:

*i*.${Ῠ}_{1}⊕{Ῠ}_{2}={Ῠ}_{2}⊕{Ῠ}_{1}$.
*ii*.${Ῠ}_{1}⊗{Ῠ}_{2}={Ῠ}_{2}⊗{Ῠ}_{1}$.
iii.$ѯ\left({Ῠ}_{1}⊕{Ῠ}_{2}\right)=ѯ{Ῠ}_{1}⊕ѯ{Ῠ}_{2}$.
*iv*.${\left({Ῠ}_{1}⊗{Ῠ}_{2}\right)}^{ѯ}={{Ῠ}_{1}}^{ѯ}⊗{{Ῠ}_{2}}^{ѯ}\text{,}$ѯ≥0.
*v*.$Ῠ⊕{ѯ}_{2}Ῠ=\left({ѯ}_{1}+{ѯ}_{2}\right)Ῠ$$,{ѯ}_{2}\geq 0$.
*vi*.${Ῠ}^{{ѯ}_{1}}⊗{Ῠ}^{{ѯ}_{2}}={Ῠ}^{{ѯ}_{1}+{ѯ}_{2}}$${ѯ}_{1},{ѯ}_{2}\geq 0$.

## 4 Spherical fuzzy Aczel Alsina Heronian mean aggregation operators

In the light of Aczel Alsina aggregation tools, we illustrate a list of new approaches based on HrM operators taking into account the SF information.

Definition 16 Let ${Ῠ}_{ҏ}=\left({₥}_{ҏ}\left(ӽ\right),{ѯ}_{ҏ}\left(ӽ\right),n_{ҏ}\left(ӽ\right)\right),ҏ=1,2,3,\ldots ,n$ be any assemblage of SFVs in R. Then, the SFAAHrM operator can be described as:

$${SFAAHrM}^{t,\varphi }\left({Ῠ}_{1},{Ῠ}_{2},\ldots ,{Ῠ}_{n}\right)={\left(\left(\frac{2}{n\left(n+1\right)}\right)\left(\overset{n}{\underset{i=1}{⊕}}\overset{n}{\underset{j=1}{⊕}}\left({Ῠ}_{i}^{t}⊗{Ῠ}_{j}^{\varphi }\right)\right)\right)}^{\frac{1}{t+\varphi }}$$

Where t,φ>0.

Theorem 2 *Let*${Ῠ}_{ҏ}=\left({₥}_{ҏ}\left(ӽ\right),{ѯ}_{ҏ}\left(ӽ\right),n_{ҏ}\left(ӽ\right)\right),ҏ=1,2,3,\ldots ,n$*be any assemblage of SFVs in*R. *Then, the SFAAHrM operator can be proved as follows*:

proof: see proof of this theorem in Appendix A.

Theorem 3 *For any collection of SFVs*${Ῠ}_{ҏ}=\left({₥}_{ҏ}\left(ӽ\right),{ѯ}_{ҏ}\left(ӽ\right),n_{ҏ}\left(ӽ\right)\right),ҏ=1,2,3,\ldots ,n$*that is*; ${Ῠ}_{n}=Ῠ$. *Then*, *we have*:

$${SFAAHrM}^{t,\varphi }\left({Ῠ}_{1},{Ῠ}_{2},\ldots ,{Ῠ}_{n}\right)=Ῠ$$

Theorem 4 *Consider*${Ῠ}_{ҏ}=\left({₥}_{ҏ}\left(ӽ\right),{ѯ}_{ҏ}\left(ӽ\right),n_{ҏ}\left(ӽ\right)\right),ҏ=1,2,3,\ldots ,n$*be the set SFVs*. *If*${Ῠ}_{ҏ}^{-}=\left\{\min\left({₥}_{ҏ}\left(ӽ\right)\right),\max\left({ѯ}_{ҏ}\left(ӽ\right)\right),\max\left(n_{ҏ}\left(ӽ\right)\right)\right\}$*and*${Ῠ}_{ҏ}^{+}=\left\{\max\left({₥}_{ҏ}\left(ӽ\right)\right),\min\left({ѯ}_{ҏ}\left(ӽ\right)\right),\min\left(n_{ҏ}\left(ӽ\right)\right)\right\}$. *Then*, *we have*:

$${Ῠ}_{ҏ}^{-}\leq SFAAHrM\left({Ῠ}_{1},{Ῠ}_{2},\ldots ,{Ῠ}_{n}\right)\leq {Ῠ}_{ҏ}^{+}$$

Theorem 5 *Let*${Ῠ}_{ҏ}\left({₥}_{ҏ}\left(ӽ\right),{ѯ}_{ҏ}\left(ӽ\right),n_{ҏ}\left(ӽ\right)\right)$*and*${Ῠ}_{ҏ}^{\prime }=\left({₥}_{ҏ}^{\prime }\left(ӽ\right),{ѯ}_{ҏ}^{\prime }\left(ӽ\right),n_{ҏ}^{\prime }\left(ӽ\right)\right),ҏ=1,2,3,\ldots ,n$*be two sets of SFVs*, *if*${Ῠ}_{ҏ}\leq {Ῠ}_{ҏ}^{\prime }$*for all*Ῠ.*Then*, *we can write as*:

$$SFAAHrM\left({Ῠ}_{1},{Ῠ}_{2},\ldots ,{Ῠ}_{n}\;\right)\leq SFAAHrM\left({Ῠ}_{1}^{\prime },{Ῠ}_{2}^{\prime },\ldots ,{Ῠ}_{n}^{\prime }\right)$$

Definition 17 Let ${Ῠ}_{ҏ}=\left({₥}_{ҏ}\left(ӽ\right),{ѯ}_{ҏ}\left(ӽ\right),n_{ҏ}\left(ӽ\right)\right),ҏ=1,2,3,\ldots ,n$ be any assemblage of SFVs in R with corresponding weight vector ${⍹}_{ҏ}$ of ${Ῠ}_{ҏ}$ such that $\sum_{ҏ=1}^{n}{⍹}_{ҏ}=1$ and ${⍹}_{ҏ}>0$. Then, the SFAAWHrM operator is described as:

$${SFAAWHrM}^{t,\varphi }\left({Ῠ}_{1},{Ῠ}_{2},\ldots ,{Ῠ}_{n}\right)={\left(ℽ\sum_{i=1}^{n}\sum_{j=1}^{n}\left({\left({⍹}_{i}{Ῠ}_{i}\right)}^{t}⊗{\left({⍹}_{j}{Ῠ}_{j}\right)}^{\varphi }\right)\right)}^{ℾ}$$

Where $ℾ=\frac{1}{t+\varphi },ℽ=\frac{2}{n\left(n+1\right)}$ and t,φ>0.

Theorem 6 *Let*${Ῠ}_{ҏ}=\left({₥}_{ҏ}\left(ӽ\right),{ѯ}_{ҏ}\left(ӽ\right),n_{ҏ}\left(ӽ\right)\right),ҏ=1,2,3,\ldots ,n$*be any assemblage of SFVs in*R*with corresponding weight vector*${⍹}_{ҏ}$*of*${Ῠ}_{ҏ}$*such that*$\sum_{ҏ=1}^{n}{⍹}_{ҏ}=1$*and*${⍹}_{ҏ}>0$. *Then*, *the SFAAWHrM operator is proved as follows*:

$${SFAAWHrM}^{t,\varphi }\left({Ῠ}_{1},{Ῠ}_{2},\ldots ,{Ῠ}_{n}\right)=\left(\begin{array}{c} e^{-{\left({ℾ\left(-\log\left(\sqrt{1-e^{-{\left(ℽ\left(\sum_{i=1}^{n}\sum_{j=1}^{n}{\left(-\log\left(1-{\left(e^{-{\left(\alpha_{i}+\alpha_{j}\right)}^{\frac{1}{₡}}}\right)}^{2}\right)\right)}^{₡}\right)\right)}^{\frac{1}{₡}}}}\right)\right)}^{₡}\right)}^{\frac{1}{₡}}},\\ \sqrt{1-e^{-{\left(ℾ{\left(-\log\left(1-{\left(e^{-{\left(ℽ\left(\sum_{i=1}^{n}\sum_{j=1}^{n}{\left(-\log\left(\sqrt{1-e^{-{\left(\beta_{i}+\beta_{j}\right)}^{\frac{1}{₡}}}}\right)\right)}^{₡}\right)\right)}^{\frac{1}{₡}}}\right)}^{2}\right)\right)}^{₡}\right)}^{\frac{1}{₡}}}},\\ \sqrt{1-e^{-{\left(ℾ{\left(-\log\left(1-{\left(e^{-{\left(ℽ\left(\sum_{i=1}^{n}\sum_{j=1}^{n}{\left(-\log\left(\sqrt{1-e^{-{\left(\gamma_{i}+\gamma_{j}\right)}^{\frac{1}{₡}}}}\right)\right)}^{₡}\right)\right)}^{\frac{1}{₡}}}\right)}^{2}\right)\right)}^{₡}\right)}^{\frac{1}{₡}}}} \end{array}\right)$$

Let

$$\alpha_{i}=\left({t\left(-\log\left(\sqrt{1-e^{-{\left({⍹}_{i}{\left(-\log\left(1-{₥}_{i}^{2}\left(ӽ\right)\right)\right)}^{₡}\right)}^{\frac{1}{₡}}}}\right)\right)}^{₡}\right)$$

$$\alpha_{j}=\left({\varphi \left(-\log\left(\sqrt{1-e^{-{\left({⍹}_{j}{\left(-\log\left(1-{₥}_{j}^{2}\left(ӽ\right)\right)\right)}^{₡}\right)}^{\frac{1}{₡}}}}\right)\right)}^{₡}\right)$$

$$\beta_{i}=\left(t{\left(-\log\left(1-{\left(e^{-{\left({{⍹}_{i}\left(-\log\left({ѯ}_{i}\left(ӽ\right)\right)\right)}^{₡}\right)}^{\frac{1}{₡}}}\right)}^{2}\right)\right)}^{₡}\right)$$

$$\beta_{j}=\left(\varphi {\left(-\log\left(1-{\left(e^{-{\left({{⍹}_{j}\left(-\log\left({ѯ}_{j}\left(ӽ\right)\right)\right)}^{₡}\right)}^{\frac{1}{₡}}}\right)}^{2}\right)\right)}^{₡}\right)$$

And

$$\gamma_{i}=\left(t{\left(-\log\left(1-{\left(e^{-{\left({{⍹}_{i}\left(-\log\left(n_{i}\left(ӽ\right)\right)\right)}^{₡}\right)}^{\frac{1}{₡}}}\right)}^{2}\right)\right)}^{₡}\right)$$

$$\gamma_{j}=\left(\varphi {\left(-\log\left(1-{\left(e^{-{\left({{⍹}_{j}\left(-\log\left(n_{j}\left(ӽ\right)\right)\right)}^{₡}\right)}^{\frac{1}{₡}}}\right)}^{2}\right)\right)}^{₡}\right)$$

For proof, move to the appendix section and see Appendix B.

Theorem 7 *For any collection of SFVs*${Ῠ}_{ҏ}=\left({₥}_{ҏ}\left(ӽ\right),{ѯ}_{ҏ}\left(ӽ\right),n_{ҏ}\left(ӽ\right)\right),ҏ=1,2,3,\ldots ,n$*that is*; ${Ῠ}_{n}=Ῠ$. *Then*, *we have*:

$${SFAAWHrM}^{t,\varphi }\left({Ῠ}_{1},{Ῠ}_{2},\ldots ,{Ῠ}_{n}\right)=Ῠ$$

Theorem 8 *Consider*${Ῠ}_{ҏ}=\left({₥}_{ҏ}\left(ӽ\right),{ѯ}_{ҏ}\left(ӽ\right),n_{ҏ}\left(ӽ\right)\right),ҏ=1,2,3,\ldots ,n$*be the set SFVs*. *If*${Ῠ}_{ҏ}^{-}=\left\{\min\left({₥}_{ҏ}\left(ӽ\right)\right),\max\left({ѯ}_{ҏ}\left(ӽ\right)\right),\max\left(n_{ҏ}\left(ӽ\right)\right)\right\}$*and*${Ῠ}_{ҏ}^{+}=\left\{\max\left({₥}_{ҏ}\left(ӽ\right)\right),\min\left({ѯ}_{ҏ}\left(ӽ\right)\right),\min\left(n_{ҏ}\left(ӽ\right)\right)\right\}$. *Then*, *we have*:

$${Ῠ}_{ҏ}^{-}\leq SFAAWHrM\left({Ῠ}_{1},{Ῠ}_{2},\ldots ,{Ῠ}_{n}\right)\leq {Ῠ}_{ҏ}^{+}$$

Theorem 9 *Let*${Ῠ}_{ҏ}\left({₥}_{ҏ}\left(ӽ\right),{ѯ}_{ҏ}\left(ӽ\right),n_{ҏ}\left(ӽ\right)\right)$*and*${Ῠ}_{ҏ}^{\prime }=\left({₥}_{ҏ}^{\prime }\left(ӽ\right),{ѯ}_{ҏ}^{\prime }\left(ӽ\right),n_{ҏ}^{\prime }\left(ӽ\right)\right),ҏ=1,2,3,\ldots ,n$*be two sets of SFVs*, *if*${Ῠ}_{ҏ}\leq {Ῠ}_{ҏ}^{\prime }$*for all*Ῠ.*Then*, *we can write as*:

$$SFAAWHrM\left({Ῠ}_{1},{Ῠ}_{2},\ldots ,{Ῠ}_{n}\;\right)\leq SFAAWHrM\left({Ῠ}_{1}^{\prime },{Ῠ}_{2}^{\prime },\ldots ,{Ῠ}_{n}^{\prime }\right)$$

## 5 Spherical fuzzy Aczel Alsina geometric heronian mean aggregation operators

Now, we derive prominent approaches of the GHrM operator based on SF information and the Aczel Alsina aggregation tools, such as SFAAGHrM and SFAAWGHrM operators.

Definition 18 Let ${Ῠ}_{ҏ}=\left({₥}_{ҏ}\left(ӽ\right),{ѯ}_{ҏ}\left(ӽ\right),n_{ҏ}\left(ӽ\right)\right),ҏ=1,2,3,\ldots ,n$ be any assemblage of SFVs in R. Then, the SFAAGHrM operator can be given as:

$$SFAAGHrM\left({Ῠ}_{1},{Ῠ}_{2},\ldots ,{Ῠ}_{n}\right)=ℾ\;\prod_{i=1}^{n}\prod_{j=1}^{n}{\left({tῨ}_{i}⊕\varphi {Ῠ}_{j}\right)}^{ℽ}$$

Where $ℾ=\frac{1}{t+\varphi },ℽ=\frac{2}{n\left(n+1\right)}$ and t,φ>0.

Theorem 10 *Let*${Ῠ}_{ҏ}=\left({₥}_{ҏ}\left(ӽ\right),{ѯ}_{ҏ}\left(ӽ\right),n_{ҏ}\left(ӽ\right)\right),ҏ=1,2,3,\ldots ,n$*be any assemblage of SFVs in*R. *Then, the SFAAGHrM operator is defined as*:

Proof: we can easily prove the above theorem.

Theorem 11 *For any collection of SFVs*${Ῠ}_{ҏ}=\left({₥}_{ҏ}\left(ӽ\right),{ѯ}_{ҏ}\left(ӽ\right),n_{ҏ}\left(ӽ\right)\right),ҏ=1,2,3,\ldots ,n$*that is*; ${Ῠ}_{n}=Ῠ$. *Then*, *we have*:

$${SFAAGHrM}^{t,\varphi }\left({Ῠ}_{1},{Ῠ}_{2},\ldots ,{Ῠ}_{n}\right)=Ῠ$$

Theorem 12 *Consider*${Ῠ}_{ҏ}=\left({₥}_{ҏ}\left(ӽ\right),{ѯ}_{ҏ}\left(ӽ\right),n_{ҏ}\left(ӽ\right)\right),ҏ=1,2,3,\ldots ,n$*be the set SFVs*. *If*${Ῠ}_{ҏ}^{-}=\left\{\min\left({₥}_{ҏ}\left(ӽ\right)\right),\max\left({ѯ}_{ҏ}\left(ӽ\right)\right),\max\left(n_{ҏ}\left(ӽ\right)\right)\right\}$*and*${Ῠ}_{ҏ}^{+}=\left\{\max\left({₥}_{ҏ}\left(ӽ\right)\right),\min\left({ѯ}_{ҏ}\left(ӽ\right)\right),\min\left(n_{ҏ}\left(ӽ\right)\right)\right\}$. *Then*, *we have*:

$${Ῠ}_{ҏ}^{-}\leq SFAAGHrM\left({Ῠ}_{1},{Ῠ}_{2},\ldots ,{Ῠ}_{n}\right)\leq {Ῠ}_{ҏ}^{+}$$

Theorem 13 *Let*${Ῠ}_{ҏ}\left({₥}_{ҏ}\left(ӽ\right),{ѯ}_{ҏ}\left(ӽ\right),n_{ҏ}\left(ӽ\right)\right)$*and*${Ῠ}_{ҏ}^{\prime }=\left({₥}_{ҏ}^{\prime }\left(ӽ\right),{ѯ}_{ҏ}^{\prime }\left(ӽ\right),n_{ҏ}^{\prime }\left(ӽ\right)\right),ҏ=1,2,3,\ldots ,n$*be two sets of SFVs*, *if*${Ῠ}_{ҏ}\leq {Ῠ}_{ҏ}^{\prime }$*for all*Ῠ.*Then*, *we can write as*:

$$SFAAGHrM\left({Ῠ}_{1},{Ῠ}_{2},\ldots ,{Ῠ}_{n}\;\right)\leq SFAAGHrM\left({Ῠ}_{1}^{\prime },{Ῠ}_{2}^{\prime },\ldots ,{Ῠ}_{n}^{\prime }\right)$$

Definition 19 Let ${Ῠ}_{ҏ}=\left({₥}_{ҏ}\left(ӽ\right),{ѯ}_{ҏ}\left(ӽ\right),n_{ҏ}\left(ӽ\right)\right),ҏ=1,2,3,\ldots ,n$ be any assemblage of SFVs in R with weight vector ${⍹}_{ҏ}$ where ҏ=1,2,3,…,n such that $\sum_{ҏ=1}^{n}{⍹}_{ҏ}=1$ and ${⍹}_{ҏ}>0$. Then, the SFAAWGHrM operator can be stated as:

$${SFAAWGHrM}^{t,\varphi }\left({Ῠ}_{1},{Ῠ}_{2},\ldots ,{Ῠ}_{n}\right)=ℾ\left(\overset{n}{\underset{i=1}{⊗}}\overset{n}{\underset{j=1}{⊗}}{\left({\left(t{Ῠ}_{i}\right)}^{{⍹}_{i}}⊕{\left(\varphi {Ῠ}_{j}\right)}^{{⍹}_{j}}\right)}^{ℽ}\right)$$

Where $ℾ=\frac{1}{t+\varphi },ℽ=\frac{2}{n\left(n+1\right)}$ and t,φ>0.

Theorem 14 *Let*${Ῠ}_{ҏ}=\left({₥}_{ҏ}\left(ӽ\right),{ѯ}_{ҏ}\left(ӽ\right),n_{ҏ}\left(ӽ\right)\right),ҏ=1,2,3,\ldots ,n$*be any assemblage of SFVs in*R*with weight vector*${⍹}_{ҏ}$*where*ҏ=1,2,3,…,n*such that*$\sum_{ҏ=1}^{n}{⍹}_{ҏ}=1$*and*${⍹}_{ҏ}>0$. *Then*, *the calculated value of the SFAAWGHrM operator is an SF value*.

$${SFAAWGHrM}^{t,\varphi }\left({Ῠ}_{1},{Ῠ}_{2},\ldots ,{Ῠ}_{n}\right)=\left(\begin{array}{c} \sqrt{1-e^{-{\left(ℾ{\left(-\log\left(1-{\left(e^{-{\left(ℽ\left(\sum_{i=1}^{n}\sum_{j=1}^{n}\left({ℽ\left(-\log\left(\sqrt{1-e^{-{\left(\alpha_{i}+\alpha_{j}\right)}^{\frac{1}{₡}}}}\right)\right)}^{₡}\right)\right)\right)}^{\frac{1}{₡}}}\right)}^{2}\right)\right)}^{₡}\right)}^{\frac{1}{₡}}}},\\ e^{-{\left({ℾ\left(-\log\left(\sqrt{1-e^{-{\left(ℽ\left(\sum_{i=1}^{n}\sum_{j=1}^{n}\left(ℽ{\left(-\log\left(1-{\left(e^{-{\left(\beta_{i}+\beta_{j}\right)}^{\frac{1}{₡}}}\right)}^{2}\right)\right)}^{₡}\right)\right)\right)}^{\frac{1}{₡}}}}\right)\right)}^{₡}\right)}^{\frac{1}{₡}}},\\ e^{-{\left({ℾ\left(-\log\left(\sqrt{1-e^{-{\left(ℽ\left(\sum_{i=1}^{n}\sum_{j=1}^{n}\left(ℽ{\left(-\log\left(1-{\left(e^{-{\left(\gamma_{i}+\gamma_{j}\right)}^{\frac{1}{₡}}}\right)}^{2}\right)\right)}^{₡}\right)\right)\right)}^{\frac{1}{₡}}}}\right)\right)}^{₡}\right)}^{\frac{1}{₡}}} \end{array}\right)$$

Where $ℾ=\frac{1}{t+\varphi },ℽ=\frac{2}{n\left(n+1\right)}$ and

let

$$\alpha_{i}={\left(-\log\left(1-{\left(e^{-{\left({{⍹}_{i}\left(-\log\left(\sqrt{1-e^{-{\left(t{\left(-\log\left(1-{₥}_{i}^{2}\left(ӽ\right)\right)\right)}^{₡}\right)}^{\frac{1}{₡}}}}\right)\right)}^{₡}\right)}^{\frac{1}{₡}}}\right)}^{2}\right)\right)}^{₡}$$

$$\alpha_{j}={\left(-\log\left(1-{\left(e^{-{\left({{⍹}_{j}\left(-\log\left(\sqrt{1-e^{-{\left(\varphi {\left(-\log\left(1-{₥}_{j}^{2}\left(ӽ\right)\right)\right)}^{₡}\right)}^{\frac{1}{₡}}}}\right)\right)}^{₡}\right)}^{\frac{1}{₡}}}\right)}^{2}\right)\right)}^{₡}$$

$$\beta_{i}={\left(-\log\left(\sqrt{1-e^{-{\left({⍹}_{i}{\left(-\log\left(1-{\left(e^{-{\left({t\left(-\log\left({ѯ}_{i}\left(ӽ\right)\right)\right)}^{₡}\right)}^{\frac{1}{₡}}}\right)}^{2}\right)\right)}^{₡}\right)}^{\frac{1}{₡}}}}\right)\right)}^{₡}$$

$$\beta_{j}={\left(-\log\left(\sqrt{1-e^{-{\left({⍹}_{j}{\left(-\log\left(1-{\left(e^{-{\left({\varphi \left(-\log\left({ѯ}_{j}\left(ӽ\right)\right)\right)}^{₡}\right)}^{\frac{1}{₡}}}\right)}^{2}\right)\right)}^{₡}\right)}^{\frac{1}{₡}}}}\right)\right)}^{₡}$$

$$\gamma_{i}={\left(-\log\left(\sqrt{1-e^{-{\left({⍹}_{i}{\left(-\log\left(1-{\left(e^{-{\left({t\left(-\log\left(n_{i}\left(ӽ\right)\right)\right)}^{₡}\right)}^{\frac{1}{₡}}}\right)}^{2}\right)\right)}^{₡}\right)}^{\frac{1}{₡}}}}\right)\right)}^{₡}$$

$$\gamma_{j}={\left(-\log\left(\sqrt{1-e^{-{\left({⍹}_{j}{\left(-\log\left(1-{\left(e^{-{\left({\varphi \left(-\log\left(n_{j}\left(ӽ\right)\right)\right)}^{₡}\right)}^{\frac{1}{₡}}}\right)}^{2}\right)\right)}^{₡}\right)}^{\frac{1}{₡}}}}\right)\right)}^{₡}$$

Proof: Proof is straightforward.

Theorem 15 *For any collection of SFVs*${Ῠ}_{ҏ}=\left({₥}_{ҏ}\left(ӽ\right),{ѯ}_{ҏ}\left(ӽ\right),n_{ҏ}\left(ӽ\right)\right),ҏ=1,2,3,\ldots ,n$*that is*; ${Ῠ}_{n}=Ῠ$. *Then*, *we have*:

$${SFAAWGHrM}^{t,\varphi }\left({Ῠ}_{1},{Ῠ}_{2},\ldots ,{Ῠ}_{n}\right)=Ῠ$$

Theorem 16 *Consider*${Ῠ}_{ҏ}=\left({₥}_{ҏ}\left(ӽ\right),{ѯ}_{ҏ}\left(ӽ\right),n_{ҏ}\left(ӽ\right)\right),ҏ=1,2,3,\ldots ,n$*be the set SFVs*. *If*${Ῠ}_{ҏ}^{-}=\left\{\min\left({₥}_{ҏ}\left(ӽ\right)\right),\max\left({ѯ}_{ҏ}\left(ӽ\right)\right),\max\left(n_{ҏ}\left(ӽ\right)\right)\right\}$*and*${Ῠ}_{ҏ}^{+}=\left\{\max\left({₥}_{ҏ}\left(ӽ\right)\right),\min\left({ѯ}_{ҏ}\left(ӽ\right)\right),\min\left(n_{ҏ}\left(ӽ\right)\right)\right\}$. *Then*, *we have*:

$${Ῠ}_{ҏ}^{-}\leq SFAAWGHrM\left({Ῠ}_{1},{Ῠ}_{2},\ldots ,{Ῠ}_{n}\right)\leq {Ῠ}_{ҏ}^{+}$$

Theorem 17 *Let*${Ῠ}_{ҏ}\left({₥}_{ҏ}\left(ӽ\right),{ѯ}_{ҏ}\left(ӽ\right),n_{ҏ}\left(ӽ\right)\right)$*and*${Ῠ}_{ҏ}^{\prime }=\left({₥}_{ҏ}^{\prime }\left(ӽ\right),{ѯ}_{ҏ}^{\prime }\left(ӽ\right),n_{ҏ}^{\prime }\left(ӽ\right)\right),ҏ=1,2,3,\ldots ,n$*be two sets of SFVs*, *if*${Ῠ}_{ҏ}\leq {Ῠ}_{ҏ}^{\prime }$*for all*Ῠ.*Then*, *we can write as*:

$$SFAAWGHrM\left({Ῠ}_{1},{Ῠ}_{2},\ldots ,{Ῠ}_{n}\;\right)\leq SFAAWGHrM\left({Ῠ}_{1}^{\prime },{Ῠ}_{2}^{\prime },\ldots ,{Ῠ}_{n}^{\prime }\right)$$

## 6 Assessment of the MADM problem based on spherical fuzzy environments

In this section, an algorithm for the MADM problem is also proposed to resolve real-life situations. We applied our invented approaches of the SFAAWHrM and SFAAWGHrM operators under the system of SF information.

Suppose that ${Ⱥ}_{\eta }=\left({Ⱥ}_{1},{Ⱥ}_{2},\ldots ,{Ⱥ}_{n}\right)$ be the set of alternatives and ${ŧ}_{ҏ}=\left({ŧ}_{1},{ŧ}_{2},\ldots ,{ŧ}_{n}\right)$ be the set of attributes with corresponding weight vectors ${⍹}_{ҏ}={\left({⍹}_{1},{⍹}_{2},\ldots ,{⍹}_{n}\right)}^{T},ҏ=1,2,3,\ldots ,n$ such that ${⍹}_{ҏ}\in \left[0,1\right]$ and $\sum_{ҏ=1}^{n}{⍹}_{ҏ}=1$. The decision maker constructed decision matrix $℟={\left(Y_{\eta ҏ}\right)}_{n\times n}$ under the system of SF information.

$$℟={\left(Y_{\eta ҏ}\right)}_{n\times n}=\left(\begin{array}{ccc} \begin{array}{c} \left({₥}_{11},{ѯ}_{11},n_{11}\right)\\ \left({₥}_{21},{ѯ}_{21},n_{21}\right)\\ \begin{array}{c} \vdots \\ \left({₥}_{n1},{ѯ}_{n1},n_{n1}\right) \end{array} \end{array} & \begin{array}{c} \left({₥}_{12},{ѯ}_{12},n_{12}\right)\\ \left({₥}_{22},{ѯ}_{22},n_{22}\right)\\ \begin{array}{c} \vdots \\ \left({₥}_{n2},{ѯ}_{n2},n_{n2}\right) \end{array} \end{array} & \begin{array}{cc} \begin{array}{c} \cdots \\ \cdots \\ \begin{array}{c} \ddots \\ \vdots \end{array} \end{array} & \begin{array}{c} \left({₥}_{1n},{ѯ}_{1n},n_{1n}\right)\\ \left({₥}_{2n},{ѯ}_{2n},n_{2n}\right)\\ \begin{array}{c} \vdots \\ \left({₥}_{nn},{ѯ}_{nn},n_{nn}\right) \end{array} \end{array} \end{array} \end{array}\right)$$

In this decision matrix, triplet $\left({₥}_{\eta ҏ},{ѯ}_{\eta ҏ},n_{\eta ҏ}\right)$ denotes the value of SFV, ${₥}_{\eta ҏ}\in \left[0,1\right]$, ${ѯ}_{\eta ҏ}\in \left[0,1\right]$ and $n_{\eta ҏ}\in \left[0,1\right]$ represent TMV, AMV, and FMV respectively. The SFV with such constraints $0\leq {₥}_{\eta ҏ}^{2}+{ѯ}_{\eta ҏ}^{2}+n_{\eta ҏ}^{2}\leq 1$. The decision maker evaluates several alternatives or individuals based on certain criteria under the system of SF information. The decision maker accumulates information on human opinions in the hypothetical form. The evaluation process of the MADM problem is based on the following steps of an algorithm.

### 6.1 Algorithm

Step 1 The decision-maker acquires SF information and states it in the decision matrix.

Step 2 The decision matrix has two types of information: beneficial and non-beneficial information. Before the evaluation of human opinions, types of information must be the same type based on the following formula:

$$℟={\left(Y_{\eta ҏ}\right)}_{n\times n}=\left\{ \begin{array}{cc} \left({₥}_{\eta ҏ},{ѯ}_{\eta ҏ},n_{\eta ҏ}\right) & \text{if}\;\text{beneficial}\;\text{factor}\\ \left(\;n_{\eta ҏ},{₥}_{\eta ҏ},{ѯ}_{\eta ҏ}\right) & \text{if}\;\text{non}-\text{beneficial}\;\text{factor} \end{array}\right.$$

Step 3 Integrate SF information to evaluate all individuals based on certain criteria. We utilized our derived strategies of the SFAAWHrM and SFAAWGHrM operators.

Step 4 To investigate suitable alternatives or individuals, compute score values using Definition 9. If the score value expression fails, we have to move on to the accuracy function.

Step 5 By rearranging the results of score values in descending order, demonstrate a suitable optimal option based on certain criteria or attributes.

### 6.2 Experimental case study

A basic human legitimate access to education is necessary to fully enjoy all other rights. It promotes personal autonomy and empowerment while also offering important development advantages. The use of comprehensive education institutes would greatly improve the quality of student learning in schools.

In Pakistan, there are several problems with the educational system. How to raise the quality of instruction in public schools is one of the largest concerns. Numerous factors contribute to this, but most people agree that the government must take a proactive approach. However, several queries and objections exist on how this would be achievable and what precisely has to be done. I'll cover the main points of it and provide some insight into the actions that must be made in order for this objective to become a reality in the essay.

Improving teacher quality must come first on the list of priorities. Better training and incentives may be given to them to do this. Additionally, the government needs to concentrate on finding more competent educators who are enthusiastic about their work rather than those who are just in education for the money. After all, teaching pupils from someone who doesn't really care about the topic or their academic achievement isn't fair. We also examined some existing models, which are prepared for the improvement of the education sector. Razzaq and Riaz [59] illustrated some new strategies based on PF information and observed how stakeholders implement new policies to improve the education sector. Sun et al. [60] explored the significance of the Internet in the field of education because advanced technologies are very useful for the system of the physical education domain. Huynh et al. [61] recommended some robust approaches for the improvement of the education sector. We also applied our invented approaches for the improvement of the education sector by using the proposed algorithm of the MADM problem.

In this experimental case study, we will study a selection process for hiring faculty members in a private university. There are several vacant posts offered. Consider five different applicants $Ⱥ=\left({Ⱥ}_{1},{Ⱥ}_{2},{Ⱥ}_{3},{Ⱥ}_{4},{Ⱥ}_{5}\right)$**,** who are shortlisted after the initial scrutiny against the vacant post of the head of the department of computer science. The panel of decision-makers evaluates the capabilities of the shortlisted applicants under certain criteria or characteristics. The selection process of applicants is completed under the following criteria.

Experience and Personality ${ŧ}_{4}-$:

Communication with students and external Public ${ŧ}_{3}-$:

Qualification and Publications ${ŧ}_{2}-$:

Management and leadership qualities ${ŧ}_{1}-$:

To evaluate information about applicants, decision-makers assign the degree of weight to the above-discussed criteria (0.15,0.20,0.35,0.30). Assessment procedure of applicants under the system of the proposed algorithm of the MADM problem.

### 6.3 Decision-making process

Evaluate the given information for improving the education sector under the SF information system. Decision makers acquire SF information in the attributes associated with each alternative. We evaluate the given information about an experimental case study by applying our derived approaches to the original information.

Step 1 The decision maker acquires SF information and lists it in the decision matrix of Table 2.

**Table 2:** Decision matrix of spherical fuzzy information.

	${ŧ}_{1}$	${ŧ}_{2}$	${ŧ}_{3}$	${ŧ}_{4}$
${Ⱥ}_{1}$	(0.67,0.34,0.41)	(0.33,0.56,0.45)	(0.66,0.5,0.38)	(0.74,0.12,0.38)
${Ⱥ}_{2}$	(0.35,0.55,0.34)	(0.65,0.34,0.51)	(0.56,0.41,0.65)	(0.65,0.41,0.56)
${Ⱥ}_{3}$	(0.45,0.36,0.47)	(0.72,0.59,0.11)	(0.45,0.7,0.3)	(0.59,0.23,0.52)
${Ⱥ}_{4}$	(0.38,0.31,0.58)	(0.21,0.70,0.58)	(0.34,0.41,0.72)	(0.29,0.49,0.69)
${Ⱥ}_{5}$	(0.39,0.56,0.41)	(0.52,0.60,0.41)	(0.27,0.67,0.58)	(0.37,0.19,0.77)

Step 2 Generally, information on the attributes is expressed in two types like: beneficial and non-beneficial. But discussed experimental case study has only beneficial information, so there is no need to transform the given decision matrix into the normalized decision matrix.

Step 3 Utilize derived approaches of the SFAAWHrM and SFAAWGHrM operators at fixed values of the t=2,φ=1, and ₡=1. Table 3 covered all investigated results by the SFAAWHrM and SFAAWGHrM operators.

**Table 3:** Aggregated results by the SFAAWHrM and SFAAWGHrM operators.

	SFAAWHrM	SFAAWGHrM
${Ⱥ}_{1}$	(0.7384,0.5313,0.5568)	(0.5461,0.7577,0.7588)
${Ⱥ}_{2}$	(0.7206,0.5610,0.5869)	(0.5353,0.7642,0.7840)
${Ⱥ}_{3}$	(0.7200,0.5665,0.5199)	(0.5352,0.7789,0.7500)
${Ⱥ}_{4}$	(0.6318,0.57120.6296)	(0.4708,0.7776,0.8059)
${Ⱥ}_{5}$	(0.6638,0.5705,0.5932)	(0.4930,0.7838,0.7910)

Step 4 Investigate score values by using Definition 9, and the obtained results are stated in Table 4. To investigate suitable alternatives, rearrange all score values in descending order. From Table 4, the raking of the score ${Ⱥ}_{1}≻{Ⱥ}_{3}≻{Ⱥ}_{2}≻{Ⱥ}_{5}≻{Ⱥ}_{4}$ is the same by the SFAAWHrM and SFAAWGHrM operators.

**Table 4:** Raking of alternatives based on computed score values from the SFAAWHrM and SFAAWGHrM operators t=2,φ=1, and ₡=1.

Operators	$k\left({Ⱥ}_{1}\right)$	$k\left({Ⱥ}_{2}\right)$	$k\left({Ⱥ}_{3}\right)$	$k\left({Ⱥ}_{4}\right)$	$k\left({Ⱥ}_{5}\right)$	Ranking and ordering
SFAAWHrM	0.6509	0.6201	0.6424	0.5588	0.5877	${Ⱥ}_{1}≻{Ⱥ}_{3}≻{Ⱥ}_{2}≻{Ⱥ}_{5}≻{Ⱥ}_{4}$
SFAAWGHrM	0.3828	0.3626	0.3724	0.3225	0.3343	${Ⱥ}_{1}≻{Ⱥ}_{3}≻{Ⱥ}_{2}≻{Ⱥ}_{5}≻{Ⱥ}_{4}$

To provide a better understanding of aggregated results, we displayed all computed results in a bar chart of Fig. 1. In Fig. 1, we clearly examine ${Ⱥ}_{1}$ is the most illegible candidate for the vacant post of the head of the department of computer science.

**Fig. 1:** Covered score values by the SFAAWHrM and SFAAWGHrM operators.

### 6.4 Influence study

This section illustrates the impact of different parametric values ₡ on the results of the SFAAWHrM and SFAAWGHrM operators. We applied different parametric values of the Aczel Alsina T-NM and TC-NM in step 3 and evaluated the results of score values. Table 5 covered the ranking of score values at fixed parametric values t=2,φ=1 and t=1,φ=1, respectively. Finally, we noted that the ranking of score values from Table 5 remains unchanged at the parametric value ₡=10**.** When taking the fixed values of t=2,φ=1 and varying the parametric values of the Aczel Alsina T-NM and TC-NM in the SFAAWHrM operator, investigated ranking of score values also shown in Table 5.

**Table 5:** Ranking of all alternatives by the SFAAWHrM operator at different parametric values of Aczel Alsina operators and some fixed variables t=2,φ=1&t=φ=1.

Parametric values	Ranking and ordering at t=2,φ=1	Ranking and ordering at t=φ=1
₡=1	${Ⱥ}_{1}≻{Ⱥ}_{3}≻{Ⱥ}_{2}≻{Ⱥ}_{5}≻{Ⱥ}_{4}$	${Ⱥ}_{1}≻{Ⱥ}_{3}≻{Ⱥ}_{2}≻{Ⱥ}_{5}≻{Ⱥ}_{4}$
₡=2	${Ⱥ}_{1}≻{Ⱥ}_{3}≻{Ⱥ}_{5}≻{Ⱥ}_{2}≻{Ⱥ}_{4}$	${Ⱥ}_{1}≻{Ⱥ}_{3}≻{Ⱥ}_{2}≻{Ⱥ}_{5}≻{Ⱥ}_{4}$
₡=5	${Ⱥ}_{1}≻{Ⱥ}_{3}≻{Ⱥ}_{2}≻{Ⱥ}_{5}≻{Ⱥ}_{4}$	${Ⱥ}_{1}≻{Ⱥ}_{3}≻{Ⱥ}_{2}≻{Ⱥ}_{5}≻{Ⱥ}_{4}$
₡=10	${Ⱥ}_{3}≻{Ⱥ}_{1}≻{Ⱥ}_{2}≻{Ⱥ}_{5}≻{Ⱥ}_{4}$	${Ⱥ}_{3}≻{Ⱥ}_{1}≻{Ⱥ}_{2}≻{Ⱥ}_{5}≻{Ⱥ}_{4}$
₡=25	${Ⱥ}_{3}≻{Ⱥ}_{1}≻{Ⱥ}_{2}≻{Ⱥ}_{5}≻{Ⱥ}_{4}$	${Ⱥ}_{3}≻{Ⱥ}_{1}≻{Ⱥ}_{2}≻{Ⱥ}_{5}≻{Ⱥ}_{4}$
₡=40	${Ⱥ}_{3}≻{Ⱥ}_{1}≻{Ⱥ}_{2}≻{Ⱥ}_{5}≻{Ⱥ}_{4}$	${Ⱥ}_{3}≻{Ⱥ}_{1}≻{Ⱥ}_{2}≻{Ⱥ}_{5}≻{Ⱥ}_{4}$
₡=55	${Ⱥ}_{3}≻{Ⱥ}_{1}≻{Ⱥ}_{2}≻{Ⱥ}_{5}≻{Ⱥ}_{4}$	${Ⱥ}_{3}≻{Ⱥ}_{1}≻{Ⱥ}_{2}≻{Ⱥ}_{5}≻{Ⱥ}_{4}$
₡=65	${Ⱥ}_{3}≻{Ⱥ}_{1}≻{Ⱥ}_{2}≻{Ⱥ}_{5}≻{Ⱥ}_{4}$	${Ⱥ}_{3}≻{Ⱥ}_{1}≻{Ⱥ}_{2}≻{Ⱥ}_{5}≻{Ⱥ}_{4}$
₡=75	${Ⱥ}_{3}≻{Ⱥ}_{1}≻{Ⱥ}_{2}≻{Ⱥ}_{5}≻{Ⱥ}_{4}$	${Ⱥ}_{3}≻{Ⱥ}_{1}≻{Ⱥ}_{2}≻{Ⱥ}_{5}≻{Ⱥ}_{4}$
₡=90	${Ⱥ}_{3}≻{Ⱥ}_{1}≻{Ⱥ}_{2}≻{Ⱥ}_{5}≻{Ⱥ}_{4}$	${Ⱥ}_{3}≻{Ⱥ}_{1}≻{Ⱥ}_{2}≻{Ⱥ}_{5}≻{Ⱥ}_{4}$
₡=100	${Ⱥ}_{3}≻{Ⱥ}_{1}≻{Ⱥ}_{2}≻{Ⱥ}_{5}≻{Ⱥ}_{4}$	${Ⱥ}_{3}≻{Ⱥ}_{1}≻{Ⱥ}_{2}≻{Ⱥ}_{5}≻{Ⱥ}_{4}$

From Table 6, we observed the results of score values at different parametric values of the Aczel Alsina aggregation tool at t=2,φ=1, and t=φ=1. After examining the results of score values and their rankings, we concluded that the raking of score values remains the same ${Ⱥ}_{1}≻{Ⱥ}_{3}≻{Ⱥ}_{2}≻{Ⱥ}_{5}≻{Ⱥ}_{4}$**.** Fig. 2, Fig. 3 covered the results of score values obtained by the SFAAWHrM operators. Fig. 4, Fig. 5 covered the graphical behavior of the SFAAWGHrM operators.

**Table 6:** Ranking of all alternatives by the SFAAWGHrM operator at different parametric values of Aczel Alsina operators and some fixed variables t=2,φ=1&t=φ=1.

Parametric values	Ranking and ordering at t=2,φ=1	Ranking and ordering at t=φ=1
₡=1	${Ⱥ}_{1}≻{Ⱥ}_{3}≻{Ⱥ}_{2}≻{Ⱥ}_{5}≻{Ⱥ}_{4}$	${Ⱥ}_{1}≻{Ⱥ}_{3}≻{Ⱥ}_{2}≻{Ⱥ}_{5}≻{Ⱥ}_{4}$
₡=2	${Ⱥ}_{1}≻{Ⱥ}_{3}≻{Ⱥ}_{2}≻{Ⱥ}_{5}≻{Ⱥ}_{4}$	${Ⱥ}_{1}≻{Ⱥ}_{3}≻{Ⱥ}_{2}≻{Ⱥ}_{5}≻{Ⱥ}_{4}$
₡=5	${Ⱥ}_{1}≻{Ⱥ}_{3}≻{Ⱥ}_{2}≻{Ⱥ}_{5}≻{Ⱥ}_{4}$	${Ⱥ}_{1}≻{Ⱥ}_{3}≻{Ⱥ}_{2}≻{Ⱥ}_{5}≻{Ⱥ}_{4}$
₡=10	${Ⱥ}_{1}≻{Ⱥ}_{3}≻{Ⱥ}_{2}≻{Ⱥ}_{5}≻{Ⱥ}_{4}$	${Ⱥ}_{1}≻{Ⱥ}_{3}≻{Ⱥ}_{2}≻{Ⱥ}_{5}≻{Ⱥ}_{4}$
₡=25	${Ⱥ}_{1}≻{Ⱥ}_{3}≻{Ⱥ}_{2}≻{Ⱥ}_{5}≻{Ⱥ}_{4}$	${Ⱥ}_{1}≻{Ⱥ}_{3}≻{Ⱥ}_{2}≻{Ⱥ}_{5}≻{Ⱥ}_{4}$
₡=40	${Ⱥ}_{1}≻{Ⱥ}_{3}≻{Ⱥ}_{2}≻{Ⱥ}_{5}≻{Ⱥ}_{4}$	${Ⱥ}_{1}≻{Ⱥ}_{3}≻{Ⱥ}_{2}≻{Ⱥ}_{5}≻{Ⱥ}_{4}$
₡=55	${Ⱥ}_{1}≻{Ⱥ}_{3}≻{Ⱥ}_{2}≻{Ⱥ}_{5}≻{Ⱥ}_{4}$	${Ⱥ}_{1}≻{Ⱥ}_{3}≻{Ⱥ}_{2}≻{Ⱥ}_{5}≻{Ⱥ}_{4}$
₡=65	${Ⱥ}_{1}≻{Ⱥ}_{3}≻{Ⱥ}_{2}≻{Ⱥ}_{4}≻{Ⱥ}_{5}$	${Ⱥ}_{1}≻{Ⱥ}_{3}≻{Ⱥ}_{2}≻{Ⱥ}_{5}≻{Ⱥ}_{4}$
₡=75	${Ⱥ}_{1}≻{Ⱥ}_{3}≻{Ⱥ}_{2}≻{Ⱥ}_{5}≻{Ⱥ}_{4}$	${Ⱥ}_{1}≻{Ⱥ}_{3}≻{Ⱥ}_{2}≻{Ⱥ}_{5}≻{Ⱥ}_{4}$
₡=90	${Ⱥ}_{1}≻{Ⱥ}_{3}≻{Ⱥ}_{2}≻{Ⱥ}_{4}≻{Ⱥ}_{5}$	${Ⱥ}_{1}≻{Ⱥ}_{3}≻{Ⱥ}_{2}≻{Ⱥ}_{5}≻{Ⱥ}_{4}$
₡=100	${Ⱥ}_{1}≻{Ⱥ}_{3}≻{Ⱥ}_{2}≻{Ⱥ}_{4}≻{Ⱥ}_{5}$	${Ⱥ}_{1}≻{Ⱥ}_{3}≻{Ⱥ}_{2}≻{Ⱥ}_{5}≻{Ⱥ}_{4}$

**Fig. 2:** Displayed the ranking of score values at t=2,φ=1.

**Fig. 3:** Displayed the raking of score values at t=φ=1.

**Fig. 4:** Displayed the raking of score values at t=2,φ=1.

**Fig. 5:** Displayed the raking of score values at t=φ=1.

## 7 Comparative study

In this discussion, we conduct a comprehensive comparative study to see the advantages and reliability of our invented approaches by applying existing strategies to the information in the literature review. We applied existing aggregation approaches seen in Refs. [57,[62], [63], [64]]. Ashraf et al. [62] gave an innovative approach by generalizing the theory of Dombi aggregation tools and resolving real-life situations. Gündoğdu and Kahraman [63] utilized basic operations of the triangular norms to illustrate the concepts of arithmetic and geometric operators under the system of SFVs. Zhang et al. [57] proposed some new strategies based on Hamacher aggregation tools to show the correctness and viability of the decision-making problem. Naeem and Ali [64] utilized some necessary operations of the Aczel Alsina aggregation tools and developed some new strategies, including SF Aczel Alsina weighted average (SFAAWA) and SF Aczel Alsina weighted geometric (SFAAWG) operators. Results obtained by the existing approaches are listed in Table 7.

**Table 7:** Aggregated outcomes from the comparative analysis.

Operators	Score values	Ranking and Ordering
SFAAWHrM	$k\left({Ⱥ}_{1}\right)≻k\left({Ⱥ}_{3}\right)≻k\left({Ⱥ}_{2}\right)≻k\left({Ⱥ}_{5}\right)≻k\left({Ⱥ}_{4}\right)$	${Ⱥ}_{1}≻{Ⱥ}_{3}≻{Ⱥ}_{2}≻{Ⱥ}_{5}≻{Ⱥ}_{4}$
SFAAWGHrM	$k\left({Ⱥ}_{1}\right)≻k\left({Ⱥ}_{3}\right)≻k\left({Ⱥ}_{2}\right)≻k\left({Ⱥ}_{5}\right)≻k\left({Ⱥ}_{4}\right)$	${Ⱥ}_{1}≻{Ⱥ}_{3}≻{Ⱥ}_{2}≻{Ⱥ}_{5}≻{Ⱥ}_{4}$
SFWA [63]	$k\left({Ⱥ}_{1}\right)≻k\left({Ⱥ}_{3}\right)≻k\left({Ⱥ}_{2}\right)≻k\left({Ⱥ}_{5}\right)≻k\left({Ⱥ}_{4}\right)$	${Ⱥ}_{1}≻{Ⱥ}_{3}≻{Ⱥ}_{2}≻{Ⱥ}_{5}≻{Ⱥ}_{4}$
SFWG [63]	$k\left({Ⱥ}_{4}\right)≻k\left({Ⱥ}_{2}\right)≻k\left({Ⱥ}_{3}\right)≻k\left({Ⱥ}_{1}\right)≻k\left({Ⱥ}_{5}\right)$	${Ⱥ}_{4}≻{Ⱥ}_{2}≻{Ⱥ}_{3}≻{Ⱥ}_{1}≻{Ⱥ}_{5}$
SFHPWA [57]	$k\left({Ⱥ}_{1}\right)≻k\left({Ⱥ}_{3}\right)≻k\left({Ⱥ}_{2}\right)≻k\left({Ⱥ}_{5}\right)≻k\left({Ⱥ}_{4}\right)$	${Ⱥ}_{1}≻{Ⱥ}_{3}≻{Ⱥ}_{2}≻{Ⱥ}_{5}≻{Ⱥ}_{4}$
SFHPWG [57]	$k\left({Ⱥ}_{4}\right)≻k\left({Ⱥ}_{2}\right)≻k\left({Ⱥ}_{3}\right)≻k\left({Ⱥ}_{1}\right)≻k\left({Ⱥ}_{5}\right)$	${Ⱥ}_{4}≻{Ⱥ}_{2}≻{Ⱥ}_{3}≻{Ⱥ}_{1}≻{Ⱥ}_{5}$
SFDWA [62]	$k\left({Ⱥ}_{1}\right)≻k\left({Ⱥ}_{3}\right)≻k\left({Ⱥ}_{2}\right)≻k\left({Ⱥ}_{5}\right)≻k\left({Ⱥ}_{4}\right)$	${Ⱥ}_{1}≻{Ⱥ}_{3}≻{Ⱥ}_{2}≻{Ⱥ}_{5}≻{Ⱥ}_{4}$
SFDWG [62]	$k\left({Ⱥ}_{1}\right)≻k\left({Ⱥ}_{4}\right)≻k\left({Ⱥ}_{2}\right)≻k\left({Ⱥ}_{3}\right)≻k\left({Ⱥ}_{5}\right)$	${Ⱥ}_{1}≻{Ⱥ}_{4}≻{Ⱥ}_{2}≻{Ⱥ}_{3}≻{Ⱥ}_{5}$
SFAAWA [64]	$k\left({Ⱥ}_{1}\right)≻k\left({Ⱥ}_{3}\right)≻k\left({Ⱥ}_{2}\right)≻k\left({Ⱥ}_{5}\right)≻k\left({Ⱥ}_{4}\right)$	${Ⱥ}_{1}≻{Ⱥ}_{3}≻{Ⱥ}_{2}≻{Ⱥ}_{5}≻{Ⱥ}_{4}$
SFAAWG [64]	$k\left({Ⱥ}_{4}\right)≻k\left({Ⱥ}_{2}\right)≻k\left({Ⱥ}_{3}\right)≻k\left({Ⱥ}_{1}\right)≻k\left({Ⱥ}_{5}\right)$	${Ⱥ}_{4}≻{Ⱥ}_{2}≻{Ⱥ}_{3}≻{Ⱥ}_{1}≻{Ⱥ}_{5}$

From Table 7, we examined the ranking of all alternatives or individuals. After evaluating the results of the existing approaches, we concluded that our invented methodologies are more applicable and efficient due to involving different parametric variables. By the variation of these parametric values and different variables, decision-makers may achieve some reliable results according to their own preferences. To better understand the significance of diagnosed mathematical approaches, we show the graphical behavior of existing approaches in a bar chart of Fig. 6.

**Fig. 6:** Shows the results of existing approaches.

## 8 Conclusions

To choose the most realistic opportunities, it is necessary to categorize various solutions. The decision-making is challenging because it differs from scene to scene. It is crucial to weigh the benefits and drawbacks of each alternative. In this article, operations of Aczel Alsina aggregation tools were developed to compile uncertain and imprecision information under the system of SF information. Numerous researchers utilized the theory of HrM operators to expose relationships among different arguments. By generalizing the concepts of HrM operators, we developed a series of new approaches based on Aczel Alsina operations, including SFAAHrM, SFAAWHrM, SFAAGHrM, and SFAAWGHrM operators. To show the reliability and consistency of our derived approaches, we expressed some appropriate characteristics of our proposed methodologies. The theory of the MAGDM problem is also illustrated to resolve daily life challenges. Utilizing an algorithm of the MAGDM technique, a practical case study was determined to select a suitable applicant for the vacant post of the head of the computer science department. We noted that ${Ⱥ}_{1}$ is the most eligible candidate for the vacant post of the head of the Department of Computer Science. Contrasting findings of proposed approaches with existing operators in the literature review express the consistency and effectiveness of our developed methodologies.

Although proposed mathematical approaches have the advantages mentioned above, it is also feasible to discuss their shortcomings. The weight of the experts or criteria must be known or at least partially known for the proposed study to address this scenario. We can derive reliable mathematical models with unknown weight to get around these restrictions for the SF circumstances. Future studies will expand on the work presented here. This effort is sure to motivate researchers and scholars to take their work in a new direction. Future work could expand the suggested methods to include linguistic data [65], bipolar complex fuzzy system [66], theory of linear diophantine fuzzy sets [67], quasirung orthopair fuzzy theory [68], 3, 4-quasirung fuzzy theory [69] and complex T-spherical fuzzy sets [70]. Moreover, the model can be integrated with the recent decision-making models [[74], [75], [76], [77], [78]]. To enhance the consistency of our derived approaches, we will apply our derived methodologies and try to resolve different applications like artificial intelligence, networking and programming, social science, waste management, and game theory. Table 8 covers all abbreviations that are used in this article.

**Table 8:** List of Abbreviations that are used in this presentation.

Abbreviation	Meanings	Abbreviation	Meanings
SFSs	spherical fuzzy sets	SF	spherical fuzzy
DMs	decision-makers	GHrM	Geometric Heronian mean
HrM	Heronian mean	FS	Fuzzy set
TMV	truth membership value	IFS	Intuitionistic fuzzy set
AMV	abstinence membership values	PyFS	Pythagorean fuzzy set
FMV	falsity membership value	q-ROFS	q-rung orthopair fuzzy set
SFAAHrM	SF Aczel Alsina Heronian mean	PFS	Picture fuzzy set
SFAAWHrM	SF Aczel Alsina weighted Heronian mean	T-SFS	T-spherical fuzzy set
SFAAGHrM	SF Aczel Alsina geometric Heronian mean (SFAAGHrM)	T-NM	t-norm
SFAAWGHrM	SF Aczel Alsina weighted geometric Heronian mean	TC-NM	t-conorm
MADM	Multi-attribute decision-making making		

## 9 Data availability

Data that has been used is confidential.

## CRediT authorship contribution statement

**Abrar Hussain:** Writing – original draft, Methodology, Formal analysis, Conceptualization. **Kifayat Ullah:** Writing – original draft, Methodology, Investigation, Formal analysis, Conceptualization. **Sajid Latif:** Writing – original draft, Methodology, Investigation, Data curation. **Tapan Senapati:** Writing – review & editing, Visualization, Validation, Investigation. **Sarbast Moslem:** Writing – review & editing, Visualization, Validation, Supervision. **Domokos Esztergar-Kiss:** Writing – review & editing, Supervision, Project administration.

## Declaration of competing interest

The authors declare that they have no known competing financial interests or personal relationships that could have appeared to influence the work reported in this paper.

## Appendix A covered the proof of Theorem 2

Let ${Ῠ}_{ҏ}=\left({₥}_{ҏ}\left(ӽ\right),{ѯ}_{ҏ}\left(ӽ\right),n_{ҏ}\left(ӽ\right)\right),ҏ=1,2,3,\ldots ,n$ be any assemblage of SFVs in R. Then,

$${Ῠ}_{i}^{t}=\left(\begin{array}{c} e^{-{\left({t\left(-\log\left({₥}_{i}\left(ӽ\right)\right)\right)}^{₡}\right)}^{\frac{1}{₡}}},\\ \sqrt{1-e^{-{\left(t{\left(-\log\left(1-{ѯ}_{i}^{2}\left(ӽ\right)\right)\right)}^{₡}\right)}^{\frac{1}{₡}}}},\\ \sqrt{1-e^{-{\left(t{\left(-\log\left(1-n_{i}^{2}\left(ӽ\right)\right)\right)}^{₡}\right)}^{\frac{1}{₡}}}} \end{array}\right)$$

$${Ῠ}_{j}^{\varphi }=\left(\begin{array}{c} e^{-{\left({\varphi \left(-\log\left({₥}_{j}\left(ӽ\right)\right)\right)}^{₡}\right)}^{\frac{1}{₡}}},\\ \sqrt{1-e^{-{\left(\varphi {\left(-\log\left(1-{ѯ}_{j}^{2}\left(ӽ\right)\right)\right)}^{₡}\right)}^{\frac{1}{₡}}}},\\ \sqrt{1-e^{-{\left(\varphi {\left(-\log\left(1-n_{j}^{2}\left(ӽ\right)\right)\right)}^{₡}\right)}^{\frac{1}{₡}}}} \end{array}\right)$$

$$\left({Ῠ}_{i}^{t}⊗{Ῠ}_{j}^{\varphi }\right)=\left(\begin{array}{c} e^{-{\left(\left({t\left(-\log\left({₥}_{i}\left(ӽ\right)\right)\right)}^{₡}\right)+\left({\varphi \left(-\log\left({₥}_{j}\left(ӽ\right)\right)\right)}^{₡}\right)\right)}^{\frac{1}{₡}}},\\ \sqrt{1-e^{-{\left(\left(t{\left(-\log\left(1-{ѯ}_{i}^{2}\left(ӽ\right)\right)\right)}^{₡}\right)+\left(\varphi {\left(-\log\left(1-{ѯ}_{j}^{2}\left(ӽ\right)\right)\right)}^{₡}\right)\right)}^{\frac{1}{₡}}}},\\ \sqrt{1-e^{-{\left(\left(t{\left(-\log\left(1-n_{i}^{2}\left(ӽ\right)\right)\right)}^{₡}\right)+\left(\varphi {\left(-\log\left(1-n_{j}^{2}\left(ӽ\right)\right)\right)}^{₡}\right)\right)}^{\frac{1}{₡}}}} \end{array}\right)$$

$$\overset{n}{\underset{j=1}{⊕}}\left({Ῠ}_{i}^{t}⊗{Ῠ}_{j}^{\varphi }\right)=\left(\begin{array}{c} \sqrt{1-e^{-{\left(\sum_{j=1}^{n}{\left(-\log\left(1-{\left(e^{-{\left(\left({t\left(-\log\left({₥}_{i}\left(ӽ\right)\right)\right)}^{₡}\right)+\left({\varphi \left(-\log\left({₥}_{j}\left(ӽ\right)\right)\right)}^{₡}\right)\right)}^{\frac{1}{₡}}}\right)}^{2}\right)\right)}^{₡}\right)}^{\frac{1}{₡}}}},\\ e^{-{\left(\sum_{j=1}^{n}{\left(-\log\left(\sqrt{1-e^{-{\left(\left(t{\left(-\log\left(1-{ѯ}_{i}^{2}\left(ӽ\right)\right)\right)}^{₡}\right)+\left(\varphi {\left(-\log\left(1-{ѯ}_{j}^{2}\left(ӽ\right)\right)\right)}^{₡}\right)\right)}^{\frac{1}{₡}}}}\right)\right)}^{₡}\right)}^{\frac{1}{₡}}},\\ e^{-{\left(\sum_{j=1}^{n}{\left(-\log\left(\sqrt{1-e^{-{\left(\left(t{\left(-\log\left(1-n_{i}^{2}\left(ӽ\right)\right)\right)}^{₡}\right)+\left(\varphi {\left(-\log\left(1-n_{j}^{2}\left(ӽ\right)\right)\right)}^{₡}\right)\right)}^{\frac{1}{₡}}}}\right)\right)}^{₡}\right)}^{\frac{1}{₡}}} \end{array}\right)$$

$$\left(\overset{n}{\underset{i=1}{⊕}}\overset{n}{\underset{j=1}{⊕}}\left({Ῠ}_{i}^{t}⊗{Ῠ}_{j}^{\varphi }\right)\right)=\left(\begin{array}{c} \sqrt{1-e^{-{\left(\sum_{i=1}^{n}\sum_{j=1}^{n}{\left(-\log\left(1-{\left(e^{-{\left(\left({t\left(-\log\left({₥}_{i}\left(ӽ\right)\right)\right)}^{₡}\right)+\left({\varphi \left(-\log\left({₥}_{j}\left(ӽ\right)\right)\right)}^{₡}\right)\right)}^{\frac{1}{₡}}}\right)}^{2}\right)\right)}^{₡}\right)}^{\frac{1}{₡}}}},\\ e^{-{\left(\sum_{i=1}^{n}\sum_{j=1}^{n}{\left(-\log\left(\sqrt{1-e^{-{\left(\left(t{\left(-\log\left(1-{ѯ}_{i}^{2}\left(ӽ\right)\right)\right)}^{₡}\right)+\left(\varphi {\left(-\log\left(1-{ѯ}_{j}^{2}\left(ӽ\right)\right)\right)}^{₡}\right)\right)}^{\frac{1}{₡}}}}\right)\right)}^{₡}\right)}^{\frac{1}{₡}}},\\ e^{-{\left(\sum_{i=1}^{n}\sum_{j=1}^{n}{\left(-\log\left(\sqrt{1-e^{-{\left(\left(t{\left(-\log\left(1-n_{i}^{2}\left(ӽ\right)\right)\right)}^{₡}\right)+\left(\varphi {\left(-\log\left(1-n_{j}^{2}\left(ӽ\right)\right)\right)}^{₡}\right)\right)}^{\frac{1}{₡}}}}\right)\right)}^{₡}\right)}^{\frac{1}{₡}}} \end{array}\right)$$

$$\left(\frac{2}{n\left(n+1\right)}\right)\left(\overset{n}{\underset{i=1}{⊕}}\overset{n}{\underset{j=1}{⊕}}\left({Ῠ}_{i}^{t}⊗{Ῠ}_{j}^{\varphi }\right)\right)=\left(\begin{array}{c} \sqrt{1-e^{-{\left(\left(\frac{2}{n\left(n+1\right)}\right)\left(\sum_{i=1}^{n}\sum_{j=1}^{n}{\left(-\log\left(1-{\left(e^{-{\left(\left({t\left(-\log\left({₥}_{i}\left(ӽ\right)\right)\right)}^{₡}\right)+\left({\varphi \left(-\log\left({₥}_{j}\left(ӽ\right)\right)\right)}^{₡}\right)\right)}^{\frac{1}{₡}}}\right)}^{2}\right)\right)}^{₡}\right)\right)}^{\frac{1}{₡}}}},\\ e^{-{\left(\left(\frac{2}{n\left(n+1\right)}\right)\left(\sum_{i=1}^{n}\sum_{j=1}^{n}{\left(-\log\left(\sqrt{1-e^{-{\left(\left(t{\left(-\log\left(1-{ѯ}_{i}^{2}\left(ӽ\right)\right)\right)}^{₡}\right)+\left(\varphi {\left(-\log\left(1-{ѯ}_{j}^{2}\left(ӽ\right)\right)\right)}^{₡}\right)\right)}^{\frac{1}{₡}}}}\right)\right)}^{₡}\right)\right)}^{\frac{1}{₡}}},\\ e^{-{\left(\left(\frac{2}{n\left(n+1\right)}\right)\left(\sum_{i=1}^{n}\sum_{j=1}^{n}{\left(-\log\left(\sqrt{1-e^{-{\left(\left(t{\left(-\log\left(1-n_{i}^{2}\left(ӽ\right)\right)\right)}^{₡}\right)+\left(\varphi {\left(-\log\left(1-n_{j}^{2}\left(ӽ\right)\right)\right)}^{₡}\right)\right)}^{\frac{1}{₡}}}}\right)\right)}^{₡}\right)\right)}^{\frac{1}{₡}}} \end{array}\right)$$

## Appendix B covered the proof of theorem 6

By using fundamental AA aggregation operations, we prove Theorem 6 as follows:

$${⍹}_{i}{Ῠ}_{i}=\left(\begin{array}{c} \sqrt{1-e^{-{\left({⍹}_{i}{\left(-\log\left(1-{₥}_{i}^{2}\left(ӽ\right)\right)\right)}^{₡}\right)}^{\frac{1}{₡}}}},\\ e^{-{\left({{⍹}_{i}\left(-\log\left({ѯ}_{i}\left(ӽ\right)\right)\right)}^{₡}\right)}^{\frac{1}{₡}}},e^{-{\left({{⍹}_{i}\left(-\log\left(n_{i}\left(ӽ\right)\right)\right)}^{₡}\right)}^{\frac{1}{₡}}} \end{array}\right)$$

$${⍹}_{j}{Ῠ}_{j}=\left(\begin{array}{c} \sqrt{1-e^{-{\left({⍹}_{j}{\left(-\log\left(1-{₥}_{j}^{2}\left(ӽ\right)\right)\right)}^{₡}\right)}^{\frac{1}{₡}}}},\\ e^{-{\left({{⍹}_{j}\left(-\log\left({ѯ}_{j}\left(ӽ\right)\right)\right)}^{₡}\right)}^{\frac{1}{₡}}},e^{-{\left({{⍹}_{j}\left(-\log\left(n_{j}\left(ӽ\right)\right)\right)}^{₡}\right)}^{\frac{1}{₡}}} \end{array}\right)$$

$${\left({⍹}_{i}{Ῠ}_{i}\right)}^{t}=\left(\begin{array}{c} e^{-{\left({t\left(-\log\left(\sqrt{1-e^{-{\left({⍹}_{i}{\left(-\log\left(1-{₥}_{i}^{2}\left(ӽ\right)\right)\right)}^{₡}\right)}^{\frac{1}{₡}}}}\right)\right)}^{₡}\right)}^{\frac{1}{₡}}},\\ \sqrt{1-e^{-{\left(t{\left(-\log\left(1-{\left(e^{-{\left({{⍹}_{i}\left(-\log\left({ѯ}_{i}\left(ӽ\right)\right)\right)}^{₡}\right)}^{\frac{1}{₡}}}\right)}^{2}\right)\right)}^{₡}\right)}^{\frac{1}{₡}}}},\\ \sqrt{1-e^{-{\left(t{\left(-\log\left(1-{\left(e^{-{\left({{⍹}_{i}\left(-\log\left(n_{i}\left(ӽ\right)\right)\right)}^{₡}\right)}^{\frac{1}{₡}}}\right)}^{2}\right)\right)}^{₡}\right)}^{\frac{1}{₡}}}} \end{array}\right)$$

$${\left({⍹}_{j}{Ῠ}_{j}\right)}^{\varphi }=\left(\begin{array}{c} e^{-{\left({\varphi \left(-\log\left(\sqrt{1-e^{-{\left({⍹}_{j}{\left(-\log\left(1-{₥}_{j}^{2}\left(ӽ\right)\right)\right)}^{₡}\right)}^{\frac{1}{₡}}}}\right)\right)}^{₡}\right)}^{\frac{1}{₡}}},\\ \sqrt{1-e^{-{\left(\varphi {\left(-\log\left(1-{\left(e^{-{\left({{⍹}_{j}\left(-\log\left({ѯ}_{j}\left(ӽ\right)\right)\right)}^{₡}\right)}^{\frac{1}{₡}}}\right)}^{2}\right)\right)}^{₡}\right)}^{\frac{1}{₡}}}},\\ \sqrt{1-e^{-{\left(\varphi {\left(-\log\left(1-{\left(e^{-{\left({{⍹}_{j}\left(-\log\left(n_{j}\left(ӽ\right)\right)\right)}^{₡}\right)}^{\frac{1}{₡}}}\right)}^{2}\right)\right)}^{₡}\right)}^{\frac{1}{₡}}}} \end{array}\right)$$

$${\left({⍹}_{i}{Ῠ}_{i}\right)}^{t}⊗{\left({⍹}_{j}{Ῠ}_{j}\right)}^{\varphi }=\left(\begin{array}{c} e^{-{\left(\alpha_{i}+\alpha_{j}\right)}^{\frac{1}{₡}}},\\ \sqrt{1-e^{-{\left(\beta_{i}+\beta_{j}\right)}^{\frac{1}{₡}}}},\\ \sqrt{1-e^{-{\left(\gamma_{i}+\gamma_{j}\right)}^{\frac{1}{₡}}}} \end{array}\right)$$

Suppose that,

$$\alpha_{i}=\left({t\left(-\log\left(\sqrt{1-e^{-{\left({⍹}_{i}{\left(-\log\left(1-{₥}_{i}^{2}\left(ӽ\right)\right)\right)}^{₡}\right)}^{\frac{1}{₡}}}}\right)\right)}^{₡}\right)$$

$$\alpha_{j}=\left({\varphi \left(-\log\left(\sqrt{1-e^{-{\left({⍹}_{j}{\left(-\log\left(1-{₥}_{j}^{2}\left(ӽ\right)\right)\right)}^{₡}\right)}^{\frac{1}{₡}}}}\right)\right)}^{₡}\right)$$

$$\beta_{i}=\left(t{\left(-\log\left(1-{\left(e^{-{\left({{⍹}_{i}\left(-\log\left({ѯ}_{i}\left(ӽ\right)\right)\right)}^{₡}\right)}^{\frac{1}{₡}}}\right)}^{2}\right)\right)}^{₡}\right)$$

$$\beta_{j}=\left(\varphi {\left(-\log\left(1-{\left(e^{-{\left({{⍹}_{j}\left(-\log\left({ѯ}_{j}\left(ӽ\right)\right)\right)}^{₡}\right)}^{\frac{1}{₡}}}\right)}^{2}\right)\right)}^{₡}\right)$$

$$\gamma_{i}=\left(t{\left(-\log\left(1-{\left(e^{-{\left({{⍹}_{i}\left(-\log\left(n_{i}\left(ӽ\right)\right)\right)}^{₡}\right)}^{\frac{1}{₡}}}\right)}^{2}\right)\right)}^{₡}\right)$$

$$\gamma_{j}=\left(\varphi {\left(-\log\left(1-{\left(e^{-{\left({{⍹}_{j}\left(-\log\left(n_{j}\left(ӽ\right)\right)\right)}^{₡}\right)}^{\frac{1}{₡}}}\right)}^{2}\right)\right)}^{₡}\right)$$

$$=\left(\begin{array}{c} e^{-{\left(\alpha_{i}+\alpha_{j}\right)}^{\frac{1}{₡}}},\\ \sqrt{1-e^{-{\left(\beta_{i}+\beta_{j}\right)}^{\frac{1}{₡}}}},\\ \sqrt{1-e^{-{\left(\gamma_{i}+\gamma_{j}\right)}^{\frac{1}{₡}}}} \end{array}\right)$$

$$\overset{n}{\underset{j=1}{⨁}}\left({\left({⍹}_{i}{Ῠ}_{i}\right)}^{t}⊗{\left({⍹}_{j}{Ῠ}_{j}\right)}^{\varphi }\right)=\left(\begin{array}{c} \sqrt{1-e^{-{\left(\sum_{j=1}^{n}{\left(-\log\left(1-{\left(e^{-{\left(\alpha_{i}+\alpha_{j}\right)}^{\frac{1}{₡}}}\right)}^{2}\right)\right)}^{₡}\right)}^{\frac{1}{₡}}}},\\ e^{-{\left(\sum_{j=1}^{n}{\left(-\log\left(\sqrt{1-e^{-{\left(\beta_{i}+\beta_{j}\right)}^{\frac{1}{₡}}}}\right)\right)}^{₡}\right)}^{\frac{1}{₡}}},\\ e^{-{\left(\sum_{j=1}^{n}{\left(-\log\left(\sqrt{1-e^{-{\left(\gamma_{i}+\gamma_{j}\right)}^{\frac{1}{₡}}}}\right)\right)}^{₡}\right)}^{\frac{1}{₡}}} \end{array}\right)$$

$$\overset{n}{\underset{i=1}{⨁}}\overset{n}{\underset{j=1}{⨁}}\left({\left({⍹}_{i}{Ῠ}_{i}\right)}^{t}⊗{\left({⍹}_{j}{Ῠ}_{j}\right)}^{\varphi }\right)=\left(\begin{array}{c} \sqrt{1-e^{-{\left(\sum_{i=1}^{n}\sum_{j=1}^{n}{\left(-\log\left(1-{\left(e^{-{\left(\alpha_{i}+\alpha_{j}\right)}^{\frac{1}{₡}}}\right)}^{2}\right)\right)}^{₡}\right)}^{\frac{1}{₡}}}},\\ e^{-{\left(\sum_{i=1}^{n}\sum_{j=1}^{n}{\left(-\log\left(\sqrt{1-e^{-{\left(\beta_{i}+\beta_{j}\right)}^{\frac{1}{₡}}}}\right)\right)}^{₡}\right)}^{\frac{1}{₡}}},\\ e^{-{\left(\sum_{i=1}^{n}\sum_{j=1}^{n}{\left(-\log\left(\sqrt{1-e^{-{\left(\gamma_{i}+\gamma_{j}\right)}^{\frac{1}{₡}}}}\right)\right)}^{₡}\right)}^{\frac{1}{₡}}} \end{array}\right)$$

$$ℽ\overset{n}{\underset{i=1}{⊕}}\overset{n}{\underset{j=1}{⊕}}\left({\left({⍹}_{i}{Ῠ}_{i}\right)}^{t}⊗{\left({⍹}_{j}{Ῠ}_{j}\right)}^{\varphi }\right)=\left(\begin{array}{c} \sqrt{1-e^{-{\left(ℽ\left(\sum_{i=1}^{n}\sum_{j=1}^{n}{\left(-\log\left(1-{\left(e^{-{\left(\alpha_{i}+\alpha_{j}\right)}^{\frac{1}{₡}}}\right)}^{2}\right)\right)}^{₡}\right)\right)}^{\frac{1}{₡}}}},\\ e^{-{\left(ℽ\left(\sum_{i=1}^{n}\sum_{j=1}^{n}{\left(-\log\left(\sqrt{1-e^{-{\left(\beta_{i}+\beta_{j}\right)}^{\frac{1}{₡}}}}\right)\right)}^{₡}\right)\right)}^{\frac{1}{₡}}},\\ e^{-{\left(ℽ\left(\sum_{i=1}^{n}\sum_{j=1}^{n}{\left(-\log\left(\sqrt{1-e^{-{\left(\gamma_{i}+\gamma_{j}\right)}^{\frac{1}{₡}}}}\right)\right)}^{₡}\right)\right)}^{\frac{1}{₡}}} \end{array}\right)$$

$${\left(ℽ\overset{n}{\underset{i=1}{⊕}}\overset{n}{\underset{j=1}{⊕}}\left({\left({⍹}_{i}{Ῠ}_{i}\right)}^{t}⊗{\left({⍹}_{j}{Ῠ}_{j}\right)}^{\varphi }\right)\right)}^{ℾ}=\left(\begin{array}{c} e^{-{\left({ℾ\left(-\log\left(\sqrt{1-e^{-{\left(ℽ\left(\sum_{i=1}^{n}\sum_{j=1}^{n}{\left(-\log\left(1-{\left(e^{-{\left(\alpha_{i}+\alpha_{j}\right)}^{\frac{1}{₡}}}\right)}^{2}\right)\right)}^{₡}\right)\right)}^{\frac{1}{₡}}}}\right)\right)}^{₡}\right)}^{\frac{1}{₡}}},\\ \sqrt{1-e^{-{\left(ℾ{\left(-\log\left(1-{\left(e^{-{\left(ℽ\left(\sum_{i=1}^{n}\sum_{j=1}^{n}{\left(-\log\left(\sqrt{1-e^{-{\left(\beta_{i}+\beta_{j}\right)}^{\frac{1}{₡}}}}\right)\right)}^{₡}\right)\right)}^{\frac{1}{₡}}}\right)}^{2}\right)\right)}^{₡}\right)}^{\frac{1}{₡}}}},\\ \sqrt{1-e^{-{\left(ℾ{\left(-\log\left(1-{\left(e^{-{\left(ℽ\left(\sum_{i=1}^{n}\sum_{j=1}^{n}{\left(-\log\left(\sqrt{1-e^{-{\left(\gamma_{i}+\gamma_{j}\right)}^{\frac{1}{₡}}}}\right)\right)}^{₡}\right)\right)}^{\frac{1}{₡}}}\right)}^{2}\right)\right)}^{₡}\right)}^{\frac{1}{₡}}}} \end{array}\right)$$

## References

[1] Zadeh L.A. (Jun. 1965). Fuzzy sets. Inf. Control.

[2] Atanassov K.T. (Oct. 1989). More on intuitionistic fuzzy sets. Fuzzy Set Syst..

[3] Yager R. (2013). 2013 Joint IFSA World Congress and NAFIPS Annual Meeting.

[4] Yager R.R. (2016). Imprecision and Uncertainty in Information Representation and Processing.

[5] Yager R.R. (Oct. 2017). Generalized orthopair fuzzy sets. Trans. Fuz Sys..

[6] Cuong B.C. (Feb. 2015). Picture fuzzy sets. JCC.

[7] Mahmood T., Ilyas M., Ali Z., Gumaei A. (2021). Spherical fuzzy sets-based cosine similarity and information measures for pattern recognition and medical diagnosis. IEEE Access.

[8] Mahmood T., Ullah K., Khan Q., Jan N. (2019). An approach toward decision-making and medical diagnosis problems using the concept of spherical fuzzy sets. Neural Comput. Appl..

[9] Ullah K., Mahmood T., Jan N. (2018). Similarity measures for T-spherical fuzzy sets with applications in pattern recognition. Symmetry.

[10] Xu Z. (2007). Intuitionistic fuzzy aggregation operators. IEEE Trans. Fuzzy Syst..

[11] Xu Z., Yager R.R. (2006). Some geometric aggregation operators based on intuitionistic fuzzy sets. Int. J. Gen. Syst..

[12] Xu Z.S., Chen J. (2008). An overview of distance and similarity measures of intuitionistic fuzzy sets. Int. J. Uncertain. Fuzziness Knowledge-Based Syst..

[13] Cerami M., Straccia U. (Jul. 2011). On the undecidability of fuzzy description logics with GCIs with Lukasiewicz t-norm. http://arxiv.org/abs/1107.4212.

[14] Aguzzoli S., Bianchi M., Valota D., Laurent A., Strauss O., Bouchon-Meunier B., Yager R.R. (2014). Information Processing and Management of Uncertainty in Knowledge-Based Systems.

[15] Lei Q., Xu Z., Bustince H., Fernandez J. (2016). Intuitionistic fuzzy integrals based on Archimedean t-conorms and t-norms. Inf. Sci..

[16] Wang W., He H. (2009). Research on flexible probability logic operator based on Frank T/S norms. ACTA ELECTONICA SINICA.

[17] Riaz M., Farid H.M.A. (2022). Multicriteria decision-making with proportional distribution based spherical fuzzy fairly aggregation operators. Int. J. Intell. Syst..

[18] Seikh M.R., Mandal U. (2023). Q-rung orthopair fuzzy archimedean aggregation operators: application in the site selection for software operating units. Symmetry.

[19] Wang J.-W. (2021). Multi-criteria decision-making method based on a weighted 2-tuple fuzzy linguistic representation model. Int. J. Inf. Technol. Decis. Making.

[20] Liu P., Li Y., Wang P. (Jan. 2023). Opinion dynamics and minimum adjustment-driven consensus model for multi-criteria large-scale group decision making under a novel social trust propagation mechanism. IEEE Trans. Fuzzy Syst..

[21] Hussain A., Ullah K., Ahmad J., Karamti H., Pamucar D., Wang H. (2022). Applications of the multiattribute decision-making for the development of the tourism industry using complex intuitionistic fuzzy hamy mean operators. Comput. Intell. Neurosci..

[22] Biswas A., Deb N. (Oct. 2021). Pythagorean fuzzy Schweizer and Sklar power aggregation operators for solving multi-attribute decision-making problems. Granul. Comput..

[23] Senapati T., Simic V., Saha A., Dobrodolac M., Rong Y., Tirkolaee E.B. (2023). Intuitionistic fuzzy power Aczel-Alsina model for prioritization of sustainable transportation sharing practices. Eng. Appl. Artif. Intell..

[24] Akram M., Naz S., Abbas T. (2023). Complex q-rung orthopair fuzzy 2-tuple linguistic group decision-making framework with Muirhead mean operators. Artif. Intell. Rev..

[25] Ali J., Naeem M. (2022). Complex q-rung orthopair fuzzy aczel–alsina aggregation operators and its application to multiple criteria decision-making with unknown weight information. IEEE Access.

[26] Akram M., Bibi R. (2023). Multi-criteria group decision-making based on an integrated PROMETHEE approach with 2-tuple linguistic Fermatean fuzzy sets. Granular Computing.

[27] Ullah K. (2021). Picture fuzzy maclaurin symmetric mean operators and their applications in solving multiattribute decision-making problems. Math. Probl Eng..

[28] Dhumras H., Bajaj R.K., Jain S., Marriwala N., Tripathi C.C., Kumar D. (2023). Emergent Converging Technologies and Biomedical Systems.

[29] Bansal P., Dhumras H., Bajaj R.K. (Nov. 2022). 2022 5th International Conference on Multimedia, Signal Processing and Communication Technologies (IMPACT).

[30] Dhumras H., Bajaj R.K. (2024). On potential strategic framework for green supply chain management in the energy sector using q-rung picture fuzzy AHP & WASPAS decision-making model. Expert Syst. Appl..

[31] Seikh M.R., Mandal U. (2021). Some picture fuzzy aggregation operators based on Frank t-norm and t-conorm: application to MADM process. Informatica.

[32] Mandal U., Seikh M.R. (Sep. 2023). Interval-valued spherical fuzzy MABAC method based on Dombi aggregation operators with unknown attribute weights to select plastic waste management process. Appl. Soft Comput..

[33] Beliakov G., Pradera A., Calvo T. (2007).

[34] Yu D. (2013). Intuitionistic fuzzy geometric Heronian mean aggregation operators. Appl. Soft Comput..

[35] Khan Q., Shahzad M., Sharif S., Elgarhy M., El-Morshedy M., Nasiru S. (2022). Applications of cubic schweizer–sklar power heronian mean to multiple attribute decision-making. Complexity.

[36] Wang H., Zhang F. (Jan. 2022). Interaction power Heronian mean aggregation operators for multiple attribute decision making with T-spherical fuzzy information. J. Intell. Fuzzy Syst..

[37] Hussain A., Ullah K., Pamucar D., Haleemzai I., Tatić D. (2023). Assessment of solar panel using multiattribute decision-making approach based on intuitionistic fuzzy Aczel Alsina heronian mean operator. Int. J. Intell. Syst..

[38] Sarkar A., Moslem S., Esztergár-Kiss D., Akram M., Jin L., Senapati T. (Sep. 2023). A hybrid approach based on dual hesitant q-rung orthopair fuzzy Frank power partitioned Heronian mean aggregation operators for estimating sustainable urban transport solutions. Eng. Appl. Artif. Intell..

[39] Li Z., Wei G. (2019). Pythagorean fuzzy heronian mean operators in multiple attribute decision making and their application to supplier selection. Int. J. Knowl. Base. Intell. Eng. Syst..

[40] Wei G., Gao H., Wei Y. (2018). Some q-rung orthopair fuzzy Heronian mean operators in multiple attribute decision making. Int. J. Intell. Syst..

[41] A. Hussain, K. Ullah, A. Al-Quran, and H. Garg, “Some T-spherical fuzzy dombi hamy mean operators and their applications to multi-criteria group decision-making process,” J. Intell. Fuzzy Syst., no. Preprint, pp. 1–21..

[42] Wei G., Lu M., Gao H. (2018). Picture fuzzy heronian mean aggregation operators in multiple attribute decision making. Int. J. Knowl. Base. Intell. Eng. Syst..

[43] Garg H., Ali Z., Gwak J., Hezam I.M. (May 2023). Generalized heronian mean operators based on archimedean T-norms of the complex picture fuzzy information and their application to decision-making. Math. Probl Eng..

[44] ur Rehman U., Mahmood T. (May 2023). A study and performance evaluation of computer network under the environment of bipolar complex fuzzy partition Heronian mean operators. Adv. Eng. Software.

[45] Hussain A., Alsanad A., Ullah K., Ali Z., Jamil M.K., Mosleh M.A. (2021). Investigating the short-circuit problem using the planarity index of complex q-rung orthopair fuzzy planar graphs. Complexity.

[46] Aczél J., Alsina C. (Dec. 1982). Characterizations of some classes of quasilinear functions with applications to triangular norms and to synthesizing judgements. Aequationes Math..

[47] Senapati T., Chen G., Mesiar R., Yager R.R. (2023). Intuitionistic fuzzy geometric aggregation operators in the framework of Aczel-Alsina triangular norms and their application to multiple attribute decision making. Expert Syst. Appl..

[48] Sarfraz M., Ullah K., Akram M., Pamucar D., Božanić D. (Dec. 2022). Prioritized aggregation operators for intuitionistic fuzzy information based on aczel–alsina T-norm and T-conorm and their applications in group decision-making. Symmetry.

[49] Hussain A., Ullah K., Alshahrani M.N., Yang M.-S., Pamucar D. (2022). Novel aczel–alsina operators for pythagorean fuzzy sets with application in multi-attribute decision making. Symmetry.

[50] Naeem M., Khan Y., Ashraf S., Weera W., Batool B. (2022). A novel picture fuzzy Aczel-Alsina geometric aggregation information: application to determining the factors affecting mango crops. AIMS Mathematics.

[51] Hussain A., Ullah K., Mubasher M., Senapati T., Moslem S. (2023). Interval-valued pythagorean fuzzy information aggregation based on Aczel-Alsina operations and their application in multiple attribute decision making. IEEE Access.

[52] Hussain A., Wang H., Ullah K., Pamucar D. (Aug. 2023). Novel intuitionistic fuzzy Aczel Alsina Hamy mean operators and their applications in the assessment of construction material. Complex Intell. Syst..

[53] Hussain A., Liu Y., Ullah K., Amjad A., Awsar A. (2023). Decision-making with unknown weights for the performance of digital devices in healthcare systems based on interval valued T-spherical fuzzy information. IEEE Access.

[54] Riaz M., Athar Farid H.M., Pamucar D., Tanveer S. (2022). Spherical fuzzy information aggregation based on aczel–alsina operations and data analysis for supply chain. Math. Probl Eng..

[55] Menger K. (1942). Statistical metrics. Proc. Natl. Acad. Sci. U.S.A..

[56] Cuong B.C. (2013).

[57] Zhang H., Wang H., Cai Q., Wei G. (2023). Spherical fuzzy hamacher power aggregation operators based on entropy for multiple attribute group decision making. J. Intell. Fuzzy Syst..

[58] Sỳkora S. (2009).

[59] Razzaq A., Riaz M. (Jan. 2023). Some modified picture fuzzy average aggregation operators with priority roles of stakeholders in implementation of education 4.0. J. Intell. Fuzzy Syst..

[60] Sun Z., Kadry S.N., Krishnamoorthy S. (Jan. 2021). Internet of things-assisted advanced dynamic information processing system for physical education system. Technol. Health Care.

[61] Huynh H.X., Nguyen L.T., Nguyen H.T., Nguyen L.T.T., Phan C.V., Nguyen T.D. (2023). Context-Aware Systems and Applications.

[62] Ashraf S., Abdullah S., Mahmood T. (2020). Spherical fuzzy Dombi aggregation operators and their application in group decision making problems. J. Ambient Intell. Hum. Comput..

[63] Kutlu Gündoğdu F., Kahraman C. (2019). Spherical fuzzy sets and spherical fuzzy TOPSIS method. J. Intell. Fuzzy Syst..

[64] Naeem M., Ali J. (2022). A novel multi-criteria group decision-making method based on Aczel–Alsina spherical fuzzy aggregation operators: application to evaluation of solar energy cells. Phys. Scripta.

[65] Akram M., Naz S., Feng F., Ali G., Shafiq A. (2023). Extended MABAC method based on 2-tuple linguistic T-spherical fuzzy sets and Heronian mean operators: an application to alternative fuel selection. AIMS Mathematics.

[66] Mahmood T., Ur Rehman U. (2022). A novel approach towards bipolar complex fuzzy sets and their applications in generalized similarity measures. Int. J. Intell. Syst..

[67] Riaz M., Hashmi M.R. (2019). Linear Diophantine fuzzy set and its applications towards multi-attribute decision-making problems. J. Intell. Fuzzy Syst..

[68] Seikh M.R., Mandal U. (Oct. 2022). Multiple attribute group decision making based on quasirung orthopair fuzzy sets: application to electric vehicle charging station site selection problem. Eng. Appl. Artif. Intell..

[69] Seikh M.R., Mandal U. (Oct. 2022). Multiple attribute decision-making based on 3,4-quasirung fuzzy sets. Granul. Comput..

[70] Ali Z., Mahmood T., Yang M.-S. (Oct. 2020). TOPSIS method based on complex spherical fuzzy sets with bonferroni mean operators. Mathematics.

[71] Kakati P., Senapati T., Moslem S., Pilla F. (2024). Fermatean fuzzy Archimedean Heronian Mean-Based Model for estimating sustainable urban transport solutions. Eng. Appl. Artif. Intell..

[72] Moslem S., Farooq D., Esztergár-Kiss D., Yaseen G., Senapati T., Deveci M. (2024). A novel spherical decision-making model for measuring the separateness of preferences for drivers' behavior factors associated with road traffic accidents. Expert Syst. Appl..

[73] Moslem S. (2024). A novel parsimonious spherical fuzzy analytic hierarchy process for sustainable urban transport solutions. Eng. Appl. Artif. Intell..

[74] Bouraima M.B., Ibrahim B., Qiu Y., Kridish M., Dantonka M. (2024). Integrated spherical decision-making model for managing climate change risks in africa. Journal of Soft Computing and Decision Analytics.

[75] Wang P., Dang R., Liu P., Pamucar D. (2023). Attitude-and cost-driven consistency optimization model for decision-making with probabilistic linguistic preference relation. Comput. Ind. Eng..

[76] Moslem S., Gündogdu F.K., Saylam S., Pilla F. (2024). A hybrid decomposed fuzzy multi-criteria decision-making model for optimizing parcel lockers location in the last-mile delivery landscape. Appl. Soft Comput..

[77] Bouraima M.B., Ibrahim B., Qiu Y., Muhammad L.J., Radovanović M. (2024). Assessment of solar energy technologies in meeting the 2030 agenda and sustainable development goals under an interval-valued fermatean fuzzy environment. Journal of Operations Intelligence.

[78] Moslem S., Deveci M., Pilla F. (2024). A novel best-worst method and Kendall model integration for optimal selection of digital voting tools to enhance citizen engagement in public decision making. Decision Analytics Journal.

